The article "Dimensional Learning Strategy-Based Grey Wolf Optimizer for Solving the Global Optimization Problem" was published in 2022. Journal: Comput Intell Neurosci.

# Dimensional Learning Strategy-Based Grey Wolf Optimizer for Solving the Global Optimization Problem

**DOI:** 10.1155/2022/3603607

**Published:** 2022-01-30

**Authors:** Xinyang Liu, Yifan Wang, Miaolei Zhou

**Affiliations:** Department of Control Science and Engineering, Jilin University, Changchun 130022, China

## Abstract

Grey wolf optimizer (GWO) is an up-to-date nature-inspired optimization algorithm which has been used for solving many of the real-world applications since it was proposed. In the standard GWO, individuals are guided by the three dominant wolves alpha, beta, and delta in the leading hierarchy of the swarm. These three wolves provide their information about the potential locations of the global optimum in the search space. This learning mechanism is easy to implement. However, when the three wolves are in conflicting directions, an individual may not obtain better knowledge to update its position. To improve the utilization of the population knowledge, in this paper, we proposed a grey wolf optimizer based on the dimensional learning strategy (DLGWO). In the DLGWO, the three dominant wolves construct an exemplar wolf through the dimensional learning strategy (DLS) to guide the grey wolves in the swarm. Thereafter, to reinforce the exploration ability of the algorithm, the Levy flight is also utilized in the proposed method. 23 classic benchmark functions and engineering problems are used to test the effectiveness of the proposed method against the standard GWO, variants of the GWO, and other metaheuristic algorithms. The experimental results show that the proposed DLGWO has good performance in solving the global optimization problems.

## 1. Introduction

tIn the real world, there are many optimization problems to be solved, and thus, the development of optimization techniques is of great importance. Most of these techniques rely on the derivatives of the functions involved in the problem, but for some reasons, derivatives of the functions are sometimes hard to obtain. As an important part of derivative-free methods, nature-inspired algorithms are attracting more and more attention for their robust searching performance. Generally, nature-inspired algorithms can be classified into three categories: evolutionary algorithms (EAs), swarm intelligence (SI), and physics-based (PB) algorithms [1–5].

SI-based algorithms, as one category of nature-inspired algorithms, are becoming increasingly popular due to their various characteristics such as strong searching ability, simple implementation, few parameters, and the ability to avoid getting trapped at local optima [6]. In these algorithms, the search agents cooperate and exchange information with each other, which guarantees that the information about the search space is efficiently utilized. This helps the whole swarm to move towards more promising area in the search space. With the progress of the algorithm, there are roughly two patterns of behavior for the swarm to perform: the exploration and the exploitation. The exploration is the process of discovering new regions of the search space. The exploitation is the process of excavating the promising area in the search space for potentially better solutions. These two patterns are conflicting [7], and maintaining an appropriate balance between them is a great challenge for any SI-based algorithm. In the past few decades, numerous SI-based algorithms have been proposed in the literature and applied to real-life problems. Some of these algorithms are very representative such as particle swarm optimization (PSO) [8], ant colony optimization (ACO) [9], artificial bee colony (ABC) algorithm [10–14], cuckoo search (CS) [15, 16], and bat algorithm (BA) [17, 18]. Some of the recent SI are teaching-learning-based optimization (TLBO) [19], salp swarm algorithm (SSA) [20], sine cosine algorithm (SCA) [21], whale optimization algorithm (WOA) [22], butterfly optimization algorithm (BOA) [23], and Harris hawks optimization (HHO) [24]. The grey wolf optimizer (GWO) was proposed by Mirjalili et al. [25] in 2014. The search mechanism of the GWO is established by mimicking the rigorous leadership hierarchy of a grey wolf pack and their group behavior when hunting. This mechanism guarantees a reliable exploration ability in the algorithm. Owing to its various advantages such as easy implementation, low computational complexity, and high search efficiency, the GWO has become quite notable and has been successfully applied to many fields in the past seven years [26, 27]. Despite the fact that the applications of the GWO technique in many fields have proved to be successful, previous works have shown that the GWO has some defects such as premature convergence and underutilization of population information and is prone to getting trapped at local optima, which are also common to some other SI-based algorithms [28, 29]. Many studies on the GWO method have been presented to address these shortcomings, which can be roughly categorized into four classes:

1. Modification of the algorithm parameters: in [30], a dynamically varying parameter *A* was adopted to maintain the proportion of wolves staying in the feasible area. In [31], Taguchi method was utilized to tune the parameters of the GWO. Rodríguez et al. [32] adopted the fuzzy inference system to dynamically adapt parameters *A* and *C*. In [33], a chaotic map was incorporated into the standard GWO to control parameters in the algorithm. Moreover, Kumar [34] provided an enhanced variant where parameter *C* was dynamically updating with the number of iterations. These modifications can improve the performance of the GWO on some problems, but the global exploration ability and local exploitation ability of the standard GWO are directly determined and balanced by the parameters *A* and *C*; thus, the modification of these parameters can break the balance between exploration and exploitation.
2. Employ novel search strategies: in [35], an enhanced GWO variant was designed based on a new wolf position update mechanism. This significantly improved the local exploitation ability of the GWO, though it might suffer from premature stagnation when dealing with multimodal problems. Cai et al. [36] introduced the random local search strategy into the standard GWO to reinforce exploration. Yang et al. [37] employed the backward learning strategy to heighten the exploration in the GWO. Despite the contributions of this work, the proposed algorithm had difficulty in solving problems with more than three objectives, and its computational consumption was higher than the standard GWO. In [38], crossover and mutation operators were incorporated into the standard GWO to improve the diversity of the population, but these operators can prevent the proposed method from converging fast. Gupta and Deep [39] modified the original GWO algorithm based on random walk. Although the proposed method cannot exhibit outstanding ability in local exploitation, the global exploration ability of the leader wolves was enhanced. In [40], the authors employed different selection methods and investigated the effects of them on the GWO. Liu et al. [41] proposed a modified GWO variant based on multiple search strategies such as the adaptive chaotic mutation strategy, boundary mutation strategy, and elitism strategy. The modified method can enhance the performance of the GWO for solving many-objective optimization problems, but it was only equipped with one type of constraint-handling technique, which might be a limitation in dealing with other practical engineering problems. In [42], the enhanced global-best lead strategy, the adaptable cooperative strategy, and the disperse foraging strategy were embedded into the GWO. Dhargupta et al. [43] combined opposition-based learning with the GWO to guarantee its exploration performance and convergence rate. Although the improvement of population diversity in the proposed algorithm is significant, it is challenging for the initial population to converge fast at the beginning of the iterations.
3. Combine with other metaheuristics: Wen et al. [44] hybridized the GWO with cuckoo search algorithm. Although there was extra computational consumption, the hybrid algorithm obtained solutions with higher quality. In [45], the GWO was combined with min-conflict algorithm. The hybrid method shows a good search performance, which can be further improved by adjusting the selection method of min-conflict algorithm. Qu et al. [46] simplified the GWO and combined it with symbiotic organisms' search. The combination of these two approaches accelerated the convergence speed of the algorithm, but individuals in the proposed method updated their positions only according to alpha, instead of the best three wolves. This put the population under the risk of trapping in the local optimum.
4. Adjustment of the hierarchy or population structure: in [47], two additional leader wolves were introduced to the leadership hierarchy to heighten the exploration ability of the standard GWO. Miao et al. [48] proposed a GWO variant based on an enhanced leading hierarchy. Yang et al. [49] divided the wolf pack into two independent groups. Fehmi Burcin Ozsoydan [50] investigated the effects of dominant wolves and made modifications to the GWO based on the variations of dominant wolves. Wang et al. [51] provided a GWO variant based on chaotic initialization. Despite the effectiveness of these adjustments, the changes in the hierarchy structure or population structure can affect the information flow mechanism of the GWO. For instance, a new leadership hierarchy might change the update process of the population, and the utilization of the multipopulation strategy might limit the utilization and exchange of information within the subpopulations.

tAccording to various works mentioned above, the main common purpose of these studies is to boost the convergence speed and accuracy of the GWO while maintaining population diversity to keep an appropriate balance between exploration and exploitation. However, the population diversity is strongly affected by the information flow mechanism of the algorithm. In the standard GWO, the search process is guided by the three dominant wolves. This leads the population to converge towards these wolves. Therefore, the information of these wolves is essential for the population, and it would reduce the search efficiency of the algorithm when the information of these wolves is conflicting.

The article "Dimensional Learning Strategy-Based Grey Wolf Optimizer for Solving the Global Optimization Problem" was published in 2022. Journal: Comput Intell Neurosci.

To improve the information utilization of the population in GWO algorithm, in this paper, the dimensional learning strategy (DLS) is implemented in the standard GWO. DLS was proposed by Xu et al. [52] to protect the potential useful information of the population best solution in PSO. In the DLS, a learning exemplar is constructed for each particle. During the constructing process, each dimension of a particle's personal best solution learns from the corresponding dimension of the population best solution. Therefore, the learning exemplar achieves the combination between the excellent information of the personal best experience and of the population best experience. Inspired by the DLS in PSO, we introduce the DLS into the leading hierarchy of GWO algorithm. There are some similarities and differences between our work and the DLS for PSO. The main purpose of employing the DLS in GWO is to efficiently protect the potential useful knowledge of the three dominant wolves, which is similar to the protection of the population best solution in PSO. The implementation of the DLS in GWO is by constructing an exemplar wolf within the three dominant wolves, which is similar to the construction of a learning exemplar between a particle's personal best solution and the population best solution in PSO. However, DLS in PSO constructs a learning exemplar for each particle based on its personal best solution and the population best solution in the current iteration. To reduce computational cost, we only construct one exemplar wolf at each iteration to guide the whole population. On each dimension, the delta wolf learns from the corresponding dimensions of both alpha and beta wolves to determine the corresponding dimension of the exemplar wolf. By employing the DLS, the potential useful knowledge of the three dominant wolves is well protected, and the situation that their information on some dimensions is conflicting is effectively avoided, which allows the GWO to utilize the knowledge of the three dominant wolves comprehensively and efficiently. In addition, to maintain an appropriate balance between exploration and exploitation, the Levy flight [15] is also employed in the algorithm. Levy flights generate steps that are drawn from the Levy distribution. Levy distribution has a good chance to randomly generate long-distance movement, which can introduce random figures to the population and improve the diversity of the population. Based on the above modifications, an enhanced grey wolf optimizer based on the dimensional learning strategy, namely, DLGWO, is proposed.

The reminder of this paper is organized as follows: the related work is introduced in Section 2. In Section 3, the proposed method is presented and illustrated in detail. Several groups of experiments to test the proposed DLGWO are conducted and reported in Section 4. In Section 5, the applications of the DLGWO to address real-world optimization problems are given. Finally, we provide the conclusion of this study in Section 6.

The article "Dimensional Learning Strategy-Based Grey Wolf Optimizer for Solving the Global Optimization Problem" was published in 2022. Journal: Comput Intell Neurosci.

## 2. Related Work

### 2.1. GWO

GWO is a metaheuristic optimization algorithm which is inspired from social hierarchy and hunting behavior of grey wolves.  Figure 1 shows the hierarchical structure in a grey wolf pack and the hunting behavior of the grey wolves in the 2D search space.

To mathematically present the social hierarchy of a wolf pack, the fittest three solutions of the population are considered as alpha (*α*), beta (*β*), and delta (*δ*), respectively. Other solutions in the population are considered as omega (*ω*).

The encircling behavior is mathematically modelled using the following equations:

(1) $$\begin{array}{c} X\left(t+1\right)=X_{\text{prey}}\left(t\right)-A\cdot B, \end{array}$$

(2) $$\begin{array}{c} B=\left|C\cdot X_{\text{prey}}\left(t\right)-X\left(t\right)\right|, \end{array}$$

(3) $$\begin{array}{c} A=2a\cdot r_{1}-a, \end{array}$$

(4) $$\begin{array}{c} C=2\cdot r_{2}, \end{array}$$

(5) $$\begin{array}{c} a=2-2\cdot \left(\frac{t}{T}\right), \end{array}$$

where *X* and *X*_prey_ are the position vectors of the wolf and the prey, respectively. *A* and *C* are coefficient vectors, and *r*_1_ and *r*_2_ are random vectors in [0,1]. *t* and *T* are the current iteration and the max iteration, respectively. The value of *a* is linearly decreasing from 2 to 0.

Assume that alpha, beta, and delta have better knowledge about the prey's position, and the other wolves update their positions according to the positions of alpha, beta, and delta. To mathematically express the hunting behavior, the equations are as follows:

(6) $$\begin{array}{c} X_{1}=\left|X_{\alpha }-A_{1}\cdot B_{\alpha }\right|,\;X_{2}=\left|X_{\beta }-A_{2}\cdot B_{\beta }\right|,\;X_{3}=\left|X_{\delta }-A_{3}\cdot B_{\delta }\right|, \end{array}$$

(7) $$\begin{array}{c} X\left(t+1\right)=\frac{X_{1}+X_{2}+X_{3}}{3}, \end{array}$$

where *X*_*α*_, *X*_*β*_, and *X*_*δ*_ are the best three solutions. *A*_1_, *A*_2_, and *A*_3_ are determined by equation (3). *B*_*α*_, *B*_*β*_, and *B*_*δ*_ are calculated using the following equations:

(8) $$\begin{array}{c} B_{\alpha }=\left|C_{1}\cdot X_{\alpha }-X\right|,\;B_{\beta }=\left|C_{2}\cdot X_{\beta }-X\right|,\;B_{\delta }=\left|C_{3}\cdot X_{\delta }-X\right|, \end{array}$$

where *C*_1_, *C*_2_, and *C*_3_ are random vectors. In the GWO, the search behavior of the grey wolves is determined by parameter *A*. Notice that *A* is generated randomly in the interval [−*a*, *a*]. |*A*| > 1 leads the search agents to expand their searching areas, and |*A*| < 1 leads the search agents to converge to the areas that have already been explored. The pseudo-code of the standard GWO is presented in Algorithm 1.

The article "Dimensional Learning Strategy-Based Grey Wolf Optimizer for Solving the Global Optimization Problem" was published in 2022. Journal: Comput Intell Neurosci.

### 2.2. PSO

PSO [8] mimics the swarm behavior, and the particles in the swarm represent search agents in the search space. Each particle updates its velocity and position by learning from its personal best position and the population best position in the search space, and the update equations are as follows:

(9) $$\begin{array}{c} v_{i,j}=wv_{i,j}+c_{1}r_{1,j}\left(x_{i,j}^{p\text{best}}-x_{i,j}\right)+c_{2}r_{2,j}\left(x_{j}^{g\text{best}}-x_{i,j}\right),\\ x_{i,j}=x_{i,j}+v_{i,j}, \end{array}$$

where *v*_*i*,*j*_ and *x*_*i*,*j*_ are the velocity and position of the *j*th dimension of particle *i*, respectively. *x*_*i*_^*p*best^ is the historical best position of particle *i*, and *x*^*g*best^ is the population historical best position. *c*_1_ and *c*_2_ are the acceleration coefficients, and *r*_1,*j*_ and *r*_2,*j*_ are two uniformly distributed random numbers independently generated in [0,1] for the *j*th dimension. The inertial weight *w* is used to control the velocity, which decreases linearly from 0.9 to 0.4 over iterations.

### 2.3. DLS for PSO

Xu et al. [52] proposed the dimensional learning strategy (DLS) to protect the potential helpful information of the particles in PSO. In the standard PSO, the particles learn from their personal best experience and population best experience. This learning strategy can lead to the phenomena of “oscillation.” [53] When the personal best position *x*_*i*_^*p*best^ and the population best position *x*^*g*best^ locate in two opposite directions of the current position *x*_*i*_, after particle *i* moves towards *x*^*g*best^, it will move closer to *x*_*i*_^*p*best^ at the next iteration since the difference *x*_*i*_^*p*best^ − *x*_*i*_ is larger than the difference *x*^*g*best^ − *x*_*i*_. A particle will constantly wander between the personal best position and the population best position, which can cause “oscillation” and limit the search efficiency of PSO. DLS is different from the learning strategy of the standard PSO. In the DLS, the personal best position *x*_*i*_^*p*best^ learns from the population best position *x*^*g*best^ dimension by dimension to construct a learning exemplar *x*_*i*_^*dl*^ which allows the excellent information of *x*^*g*best^ to be inherited by the exemplar *x*_*i*_^*dl*^, improving the information utilization of *x*^*g*best^. By replacing *x*_*i*_^*p*best^ by *x*_*i*_^*dl*^ in equation (9) of the standard PSO, the improved velocity update equation is as follows:

(10) $$\begin{array}{c} v_{i,j}=wv_{i,j}+c_{1}r_{1,j}\left(x_{i,j}^{dl}-x_{i,j}\right)+c_{2}r_{2,j}\left(x_{j}^{g\text{best}}-x_{i,j}\right). \end{array}$$

The process of constructing an exemplar *x*_*i*_^*dl*^ is shown in Algorithm 2.

The article "Dimensional Learning Strategy-Based Grey Wolf Optimizer for Solving the Global Optimization Problem" was published in 2022. Journal: Comput Intell Neurosci.

## 3. The Proposed Method

### 3.1. Motivation of the Work

In the standard GWO, other wolves update their positions according to the three dominant wolves in the leading hierarchy. These three wolves provide their information about the potential location of the prey, and their positions are closer to the global optimum or local optimum in the search space. However, when alpha, beta, and delta are located in conflicting directions, an individual may not obtain better knowledge about the promising area, as demonstrated in Figure 2. Thus, it is of great importance to protect the potential helpful knowledge of the leading hierarchy and improve the information utilization of the population.

## 4. DLS for the GWO

Inspired by the DLS in PSO [52], in this paper, DLS is employed in the leading hierarchy of the GWO to protect the potential helpful knowledge about the prey's location and guide the individuals with more efficiency. In the DLS, delta learns from both alpha and beta dimension by dimension to construct an exemplar wolf; in this way, the excellent information of the three wolves can be passed to the exemplar wolf and other wolves in the pack.  Figure 3 illustrates the process of the DLS; suppose that 4D sphere function *f*(*x*)=*x*_1_^2^+*x*_2_^2^+*x*_3_^2^+*x*_4_^2^ is the objective function of the minimum problem, which has the global minimum point (0,0,0,0)^*T*^. *X*_*α*_=(1,2,2,2)^*T*^, *X*_*β*_=(2,4,1,3)^*T*^, and *X*_*δ*_=(3,0,3,4)^*T*^ are the positions of alpha, beta, and delta, respectively. The numbers filled in red, blue, green, and yellow are the values of the three dominant wolves and the exemplar wolf at the first, second, third, and forth dimension, respectively. Initially, let the position vector of the exemplar wolf *X*_*L*_=*X*_*δ*_=(3,0,3,4)^*T*^; it is easy to calculate that *f*(*X*_*L*_)=*f*(*X*_*δ*_)=34; then, two temporary vectors *X*^temp1^ and *X*^temp2^ are set for *X*_*L*_ at each dimension during the process of the DLS which can be expressed as follows:

1. For dimension 1: let *X*_1_^temp1^=*X*_*α*,1_=1, *X*_1_^temp2^=*X*_*β*,1_=2, *X*^temp1^=(1,0,3,4)^*T*^, and *X*^temp2^=(2,0,3,4)^*T*^. *f*(*X*^temp1^)=26〈*f*(*X*^temp2^)=29〈*f*(*X*_*L*_)=34; thus, *X*_*L*,1_=*X*_1_^temp1^=1, *X*_*L*_=(1,0,3,4)^*T*^, and *f*(*X*_*L*_)=26.
2. For dimension 2: let *X*_2_^temp1^=*X*_*α*,2_=2, *X*_2_^temp2^=*X*_*β*,2_=4, *X*^temp1^=(1,2,3,4)^*T*^, and *X*^temp2^=(1,4,3,4)^*T*^. *f*(*X*_*L*_)=26〈*f*(*X*^temp1^)=30〈*f*(*X*^temp2^)=42; thus, *X*_*L*,2_ remains unchanged, *X*_*L*_=(1,0,3,4)^*T*^, and *f*(*X*_*L*_)=26.
3. For dimension 3: let *X*_3_^temp1^=*X*_*α*,3_=2, *X*_3_^temp2^=*X*_*β*,3_=1, *X*^temp1^=(1,0,2,4)^*T*^, and *X*^temp2^=(1,0,1,4)^*T*^. *f*(*X*^temp2^)=18〈*f*(*X*^temp1^)=21〈*f*(*X*_*L*_)=26; thus, *X*_*L*,3_=*X*_3_^temp2^=1, *X*_*L*_=(1,0,1,4)^*T*^, and *f*(*X*_*L*_)=18.
4. For dimension 4: let *X*_4_^temp1^=*X*_*α*,4_=2, *X*_4_^temp2^=*X*_*β*,4_=3, *X*^temp1^=(1,0,1,2)^*T*^, and *X*^temp2^=(1,0,1,3)^*T*^. *f*(*X*^temp1^)=6〈*f*(*X*^temp2^)=11〈*f*(*X*_*L*_)=18; thus, *X*_*L*,4_=*X*_4_^temp1^=2, *X*_*L*_=(1,0,1,2)^*T*^, and *f*(*X*_*L*_)=6.

The article "Dimensional Learning Strategy-Based Grey Wolf Optimizer for Solving the Global Optimization Problem" was published in 2022. Journal: Comput Intell Neurosci.

After the DLS, *X*_*L*_=(1,0,1,2)^*T*^, and it learns from alpha at the first and the forth dimensions, beta at the third dimension, and delta at the second dimension. Hence, the final *X*_*L*_ is constructed by combining *X*_*δ*_ with the dimensions learned from *X*_*α*_ and *X*_*β*_, which indicates that the exemplar wolf is not worse than the three dominant wolves. To implement the DLS in the GWO, we substitute the best three wolves in the standard GWO with the exemplar wolf to update the positions of other wolves. The improved equation is given by

(11) $$\begin{array}{c} X\left(t+1\right)=X_{L}-A_{L}\cdot B_{L},\;B_{L}=\left|C_{L}\cdot X_{L}-X\right|, \end{array}$$

where *X* is the position vector of a wolf. *X*_*L*_ is the position vector of the exemplar wolf. *B*_*L*_ is an intermediate variable. *A*_*L*_ and *C*_*L*_ can be obtained by equations (3) and (4), respectively. As illustrated by Figure 3, before the value of the exemplar wolf at the current dimension is updated, *X*_*L*_ is compared with the two temporary vectors *X*^temp1^ and *X*^temp2^. *X*^temp1^ and *X*^temp2^ are set by substituting the value of *X*_*L*_ with the value of *X*_*α*_ and *X*_*β*_ at the current dimension, respectively. If *X*^temp1^ or *X*^temp2^ is better than the exemplar wolf, the value of the exemplar wolf at the current dimension is updated. Otherwise, the exemplar wolf remains unchanged and continues the process of DLS at the next dimension. Therefore, the exemplar wolf learns only from the dimensions of the three dominant wolves that can help improve its fitness value, which guarantees that the exemplar wolf will not be degraded when alpha, beta, and delta are located in conflicting directions and hence improves the utilization of the population knowledge. The flowchart of the DLS is illustrated in Figure 4.

### 4.1. Trial Solutions Based on Levy Flight

For a SI-based algorithm, exploration and exploitation are performed simultaneously. Exploration is to discover more promising areas in the search space, and exploitation is to focus on the current optimal areas. Hence, it is important to keep an appropriate balance between exploration and exploitation. In the DLS, each grey wolf learns from the exemplar wolf; this leads the population to converge to the exemplar wolf which strengthens the exploitation ability of the algorithm and potentially causes premature convergence as well. To improve the exploration performance of the algorithm, the method proposed by Mantegna [54] to generate the Levy flight is utilized in the algorithm. In comparison to the Gaussian distribution which always generates small steps, the Levy distribution can occasionally generate long steps which is helpful for the exploration. The 2D and 3D trajectories drawn from the Levy distribution are illustrated in Figure 5.

The article "Dimensional Learning Strategy-Based Grey Wolf Optimizer for Solving the Global Optimization Problem" was published in 2022. Journal: Comput Intell Neurosci.

After a wolf updates its position according to the exemplar wolf by equation (12), a trial solution is obtained by Levy flight using the following formula:

(12) $$\begin{array}{c} X_{\text{trial}}\left(t+1\right)=X\left(t+1\right)+G\times \text{Levy}\left(D\right), \end{array}$$

where *D* is the dimension size, *G* is a randomly generated vector with the size of 1 × *D*, and Levy is the Levy flight function, which is given by

(13) $$\begin{array}{c} \text{Levy}=0.01\times \frac{u\times \phi }{{\left|v\right|}^{1/z}}, \end{array}$$

where *u* and *v* are random values in the interval [0,1] and *z* is a constant set to 1.5. *ϕ* can be expressed as

(14) $$\begin{array}{c} \phi ={\left\{\frac{\Gamma \left(1+z\right)\times \;\sin\left(\pi z/2\right)}{\Gamma \left(\left(1+z\right)/2\right)\times z\times 2^{\left(z-1\right)/2}}\right\}}^{1/z}. \end{array}$$

Then, the objective function value of the trial position *f*(*X*_trial_(*t*+1)) is compared with that of the updated position *f*(*X*(*t*+1)), and the position with the smaller value is preserved, which can be expressed by

(15) $$\begin{array}{c} X\left(t+1\right)=\left\{\begin{array}{cc} X\left(t+1\right) & \text{if }f\left(X\left(t+1\right)\right)\leq f\left(X_{\text{trial}}\left(t+1\right)\right),\\ X_{\text{trial}}\left(t+1\right) & \text{if }f\left(X\left(t+1\right)\right)>f\left(X_{\text{trial}}\left(t+1\right)\right). \end{array}\right. \end{array}$$

### 4.2. The Proposed DLGWO Algorithm

By employing the DLS and Levy flight, we proposed an enhanced variant of the GWO, named as dimension learning grey wolf optimizer (DLGWO). The framework of the proposed DLGWO is illustrated in Figure 6. Firstly, DLS is utilized to protect the potential useful knowledge of the three dominant wolves; this enhances search efficiency and reinforces the exploitation ability simultaneously. Secondly, Levy flight is embedded into the algorithm as an effective measure to guarantee population diversity and strengthen the exploration ability. The process of constructing the exemplar wolf is shown in Algorithm 3.

The article "Dimensional Learning Strategy-Based Grey Wolf Optimizer for Solving the Global Optimization Problem" was published in 2022. Journal: Comput Intell Neurosci.

### 4.3. Analysis of Computational Complexity

The computational costs of the standard GWO include initialization *O*(*n*  *D*), evaluation at each iteration *O*(*n*), selecting the dominant wolves *O*(*n*), and position updating *O*(*n*  *D*); *n* and *D* are the population and dimension size, respectively. For the DLGWO, the additional costs occur when the dimensional learning process is utilized in which the position vector of the exemplar wolf is constructed by comparing *f*(*X*_*L*_) with the smaller value of *f*(*X*^temp1^) and *f*(*X*^temp2^), and since the position vector of the exemplar wolf has been updated and recorded during the process, the employing of the DLS requires additional computation of 2  *D* fitness evaluations *O*(2  *D*) in each iteration. From the above analysis, the computational complexity for the standard GWO and DLGWO is at the same level.

## 5. Experimental Verification and Analysis

In this section, 4 experiments are carried out and presented. First, the efficacy of the DLS and Levy flight in the proposed algorithm is verified. Then, we perform experiments to verify the capacity of the DLGWO on functions of different dimensions. After that, the proposed DLGWO is compared with the GWO and its 6 promising variants. Finally, DLGWO is examined with other well-established metaheuristics. A widely utilized set of benchmark functions is employed [28, 30, 40, 48, 55], and the detailed information about the benchmark functions can be found in Table 1. As presented in Table 1, the test set includes 7 unimodal functions (*f*1–*f*7), 6 multimodal functions (*f*8–*f*13), and 10 fixed-dimension multimodal functions (*f*14–*f*23). There is only one global optimal solution in unimodal functions; thus, these functions are suitable for evaluating the local exploitation capability of an algorithm. With respect to the multimodal functions, they have several local optimal solutions besides the global optimal solution and thus are utilized to challenge the global exploration ability and the capacity of avoiding the local optimum. The fixed-dimension multimodal functions are composed of global optimum, local optimum, and many different characteristics such as rotation and shift and are used to examine the ability of an algorithm when disposing of complicated cases.  Figure 7 demonstrates the landscapes of three benchmark functions. The indexes for comparing include the mean values (Mean), the standard deviations (SD), and rank (Rank) of the average best result for each method. Besides, to check if the improvements of the DLGWO over the other algorithms are significant, the Wilcoxon rank-sum tests at a 0.05 significance level are also utilized. The Wilcoxon rank-sum test is a paired test that checks for significant differences between two algorithms, where “+/≈/−” means that the proposed algorithm is significantly better, similar to, or significantly worse than the comparison algorithm. In addition, all the experiments are implemented using MATLAB R2016a and are run on a CPU Core i5-4210U, 4GB RAM, with Windows 10 operating system.

The article "Dimensional Learning Strategy-Based Grey Wolf Optimizer for Solving the Global Optimization Problem" was published in 2022. Journal: Comput Intell Neurosci.

### 5.1. Effect of Different Strategies

Before comprehensive evaluations, it is essential to investigate the effect of each strategy on the performance of the proposed algorithm. As mentioned above, the DLGWO algorithm consists of two main improvement strategies: DLS and Levy flight. In this part, the effectiveness of these two strategies is validated. For this purpose, a comparison between the DLGWO and its variants is conducted. Herein, its variants are denoted as the DLSGWO and LFGWO, respectively. The algorithm adopting the DLS while the Levy flight is ignored is denoted as DLSGWO. The algorithm employing the Levy flight while the DLS is not utilized is denoted as LFGWO.

To more intuitively measure the exploration and exploitation abilities of the DLGWO and its variants, we compare the search history, trajectories of the first search agent at the first dimension, and population diversity of the DLGWO, DLSGWO, LFGWO, and the standard GWO. The population diversity is calculated using the following equations:

(16) $$\begin{array}{c} \text{diversity}=\frac{1}{N}\sum_{i=1}^{N}\sqrt{\sum_{j=1}^{D}{\left(x_{i,j}-\bar{x_{j}}\right)}^{2}},\\ \bar{x_{j}}=\frac{\sum_{i=1}^{N}x_{i,j}}{N}, \end{array}$$

where *N* is the population size, *D* is the dimension of the search space, *x*_*i*,*j*_ denotes the *j*th dimension of the *i*th particle, and *x*_*j*_ denotes the *j*th dimension of the center position of the population.

The obtained results are exhibited in Figure 8. These results record the search history, trajectories of the first search agent at its first dimension, and diversity of solutions based on 20 search agents with the maximum number of function evaluations of 30000 in dealing with two unimodal functions (*f*1 and *f*2) and two multimodal functions (*f*10 and *f*11) from Table 1. The search history and trajectories are displayed in two dimensions, more clearly. These plots are recorded in the same way demonstrated in the original work of the GWO.

From the search history and trajectory plots in Figure 8, it can be seen that the DLGWO and LFGWO exhibit a better distributed scatter plot in the initial stage of iteration compared with the DLSGWO. These two methods have more extensive coverage on those unexplored areas in the search space that has not been covered efficiently by the DLSGWO. Those blue and yellow points away from the center of the search space are generated mostly based on Levy flight. Then, after initial iterations, search agents are guided towards areas with more high-quality solutions (in these four functions, the global optimum is at the center of the search space). In this process, the exemplar wolf constructed in the DLSGWO carries the information about potential areas with excellent solutions and leads the population to the center and its surrounding areas. Therefore, more search agents in the population are guided by the DLSGWO than other methods towards the vicinity of the center. This verifies the exploitation ability of the DLSGWO. By contrast, LFGWO cannot guarantee strong exploitation in further iterations; it shows a lower concentration of solutions around the optimum due to the randomness from Levy flight. Furthermore, DLGWO is able to obtain a fine balance: it exhibits a strong exploration capacity in the initial iterations and a good exploitation capacity in further iterations. This is because of the incorporation of the two strategies. As for the diversity curves in Figure 8, LFGWO obtains the highest diversity, and DLGWO is ranked second. From the results of diversity, it can be observed that the DLSGWO maintains the smallest diversity and, consequently, has high convergence speed. As expected, the LFGWO maintains the highest diversity during the initial stage, and then Levy flight can significantly improve the exploration of the search space which provides a wide range of variety in solutions. Finally, the diversity of the DLGWO is lower than that of the LFGWO, but higher than that of the standard GWO and DLSGWO. This is because of the appropriate balance between exploitation and exploration provided by the interaction and cooperation of the DLS and Levy flight. Therefore, the diversity comparison results also verify our expectation that the DLS is mainly responsible for local exploitation while Levy flight for global exploration. According to the results and analysis above, the incorporation of the DLS and Levy flight can effectively improve the balance between the exploratory and exploitative performance of the DLGWO, while the DLSGWO and LFGWO with only one of those strategies cannot obtain a better balance, individually.

The article "Dimensional Learning Strategy-Based Grey Wolf Optimizer for Solving the Global Optimization Problem" was published in 2022. Journal: Comput Intell Neurosci.

To further investigate the utility and efficacy of the DLS and Levy flight, we compare the optimization results on *f*_1_ − *f*_13_ of the DLGWO with both DLS and Levy flight, DLSGWO with the DLS alone, and LFGWO with Levy flight alone. The maximum number of fitness evaluations is set to 300000.  Table 2 presents the statistical results of unimodal functions (*f*_1_ − *f*_7_) and multimodal functions (*f*_8_ − *f*_13_), respectively. From the numerical results shown in Table 2, DLSGWO ranks first, followed by DLGWO and LFGWO, for unimodal functions; LFGWO ranks first, followed by DLGWO and DLSGWO, for multimodal functions. It can be drawn from the experimental results that DLS guarantees, in each generation, the outstanding information of the three dominant wolves to be inherited by each wolf in the swarm through the exemplar wolf, which strongly enhances the convergence performance. However, the diversity of the DLSGWO is relatively low and is easily trapped in the local optimum; thus, it is challenging for the DLS to deal with multimodal functions. Levy flight improves the diversity of the population and exhibits better performance for solving multimodal functions with many local optima. Our design expectation is verified by the experimental results that the DLS concentrates on local exploitation, while Levy flight focuses on global exploration. It is the interaction and cooperation of DLS and Levy flight that enables the competitive performance of the DLGWO for both unimodal and multimodal functions.

### 5.2. The Impact of Problem Dimension

Any efficient optimizer should be able to make a fine tradeoff between minimizing cost and maximizing accuracy. From the analysis of computational complexity, the computational cost of utilizing DLS increases as the dimension of the problem increases. To better evaluate the impact of dimension on the performance of the proposed method, DLGWO and the standard GWO are implemented on *f*_1_ − *f*_13_ from Table 1 with dimensions of 10, 30, 100, and 200. All conditions are the same, and the maximum number of fitness evaluations is 300000. By increasing the dimension, the statistical results are recorded and shown in Table 3. The boldface in Table 3 indicates the best experimental results. It can be seen from Table 3 that DLGWO outperforms the standard GWO in all dimensions with a promising and stable performance. When dimension increases, the exemplar wolf has a more comprehensive knowledge of population information at different dimensions; thus, the exemplar wolf can guide the swarm with more efficiency. However, it can also be observed that, compared with the proposed method, the standard GWO can obtain optimization results with higher accuracy on *f*_3_, *f*_5_, and *f*_13_ when the dimension increases to 200. The reason is that the extra fitness evaluations for DLGWO algorithm will also increase as the dimension rises, which can limit the performance of the DLGWO. Therefore, it is still an interesting and challenging future work to decrease the extra cost of constructing the exemplar wolf and obtain a better tradeoff between algorithm performance and computational cost.

The article "Dimensional Learning Strategy-Based Grey Wolf Optimizer for Solving the Global Optimization Problem" was published in 2022. Journal: Comput Intell Neurosci.

### 5.3. Comparison of the DLGWO with the GWO and Its Variants

In this section, the proposed DLGWO is compared with the GWO and its several promising variants. The explanations and parameter settings for these GWO variants are given in Table 4. The test functions utilized in this part are all classical benchmark problems from Table 1. Each problem is independently executed 30 times, where the number of search agents and the maximum number of fitness evaluations are 40 and 300000, respectively. The statistical results are provided in Tables 5–9.

### 5.4. Algorithm Accuracy Analysis

The numerical results on unimodal functions (*f*_1_–*f*_7_) are presented in Table 5. As for unimodal functions *f*_1_–*f*_7_, these problems are suitable for testing the exploitation ability of algorithms. From the obtained results, DLGWO achieves the best rank for *f*_1_, *f*_2_, *f*_5_, and *f*_7_. On *f*_3_, IGWO is the best optimizer with a competitive accuracy of 8.42*E* − 192, whereas DLGWO takes the second place with an accuracy of 6.53*E* − 182. On *f*_4_, DLGWO is not as competitive as GWOCS, MGWO, and IGWO and comes in the fourth place. The global optimum of *f*_5_ is in a narrow area, which is quite challenging to obtain for most optimizers; thus, the results of the DLGWO and the other algorithms for *f*_5_ are satisfactory. On *f*_6_, RWGWO exhibits slightly higher search accuracy compared with the DLGWO, but DLGWO also provides an outstanding accuracy of 4.28*E* − 07. In the final average rank, DLGWO is the best optimizer with the best exploitation ability, followed by IGWO, GWOCS, MGWO, learnGWO, SOGWO, RWGWO, and GWO.

The numerical results on multimodal functions (*f*_8_–*f*_13_) are presented in Table 6. Contrast to unimodal functions, multimodal functions are suitable for examining the exploration ability since most of them contain numerous local optima, which may lead to premature convergence of optimizers. On *f*_8_, it is difficult for the standard GWO to locate the global optimum. The reason is that this problem has many deep local optima far away from the global optima; once alpha, beta, and delta in the standard GWO are all trapped into a deep local optimum, they can hardly escape and may lead more search agents into the local optimum. From Table 6, DLGWO exhibits better ability of avoiding the local optimum and hence obtains a higher search accuracy of −8.35*E* + 03. This can be ascribed to the Levy flight strategy in the DLGWO which improves the population diversity of the algorithm. All the methods can locate the global optimum for *f*_9_ and *f*_11_. On *f*_10_, IGWO obtains the highest accuracy of 4.44*E* − 15, followed by DLGWO with an accuracy of 4.94*E* − 15. On *f*_11_, DLGWO has an apparent advantage compared with the other GWO variants, with an excellent accuracy of 1.75*E* − 08. On *f*_13_, DLGWO takes the first place, and RWGWO also obtains a competitive accuracy of 3.57*E* − 07. On multimodal problems, DLGWO also exhibits the best performance, and RWGWO is the second competitive method, followed by IGWO, learnGWO, SOGWO, GWOCS, MGWO, and GWO. As observed in the results of unimodal and multimodal functions, DLGWO obtains the best rank for 9 out of 13 problems and can achieve the global optima for 4 problems, i.e., *f*_1_, *f*_2_, *f*_9_, and *f*_11_. It ranks first statistically among all the algorithms on both unimodal and multimodal functions, which demonstrates the efficiency of the DLS and Levy flight and the strength of their interaction and cooperation.

The article "Dimensional Learning Strategy-Based Grey Wolf Optimizer for Solving the Global Optimization Problem" was published in 2022. Journal: Comput Intell Neurosci.

Table 7 presents the numerical results on the fixed-dimension multimodal functions (*f*_14_–*f*_23_). These functions can evaluate the efficiency of the algorithms when dealing with functions with different characteristics such as rotation and shift. From the results provided in Table 7, DLGWO performs best on 4 out of 10 functions, i.e., *f*_15_, *f*_16_, *f*_18_, and *f*_23_. On *f*_14_, *f*_17_, *f*_19_, *f*_21_, and *f*_22_, DLGWO has the same search accuracy compared with the algorithms ranking first (RWGWO for *f*_14_, *f*_17_, and *f*_21_, SOGWO for *f*_19_, and MGWO for *f*_22_), but DLGWO is not as robust as these algorithms and has a higher standard deviation. On *f*_20_, SOGWO obtains the global optimum, followed by DLGWO with a search accuracy of −3.28*E* + 00. On *f*_23_, DLGWO has the most robust performance with the smallest standard deviation of 5.04*E* − 07. In general, DLGWO shows competitive and robust performance on the fixed-dimensional functions, which proves that the two strategies implemented in the DLGWO show different effectiveness when dealing with functions with different features.

Tables 8 and 9 give the overall Wilcoxon rank-sum test results of the DLGWO and each algorithm. From Table 9, DLGWO outperforms the other comparative methods in different problems and obtains results of 20/3/0 vs. GWO, 14/6/3 vs. RWGWO, 19/4/0 vs. learnGWO, 18/4/1 vs. GWOCS, 14/6/3 vs. IGWO, 18/4/1 vs. SOGWO, and 16/5/2 vs. MGWO.

### 5.5. Convergence Behavior Analysis

To compare the convergence behavior, Figures 9 and 10 present the convergence curves of the DLGWO and other algorithms on *f*_1_–*f*_13_. It can be detected that the DLGWO has the fastest convergence speed on *f*_1_ and *f*_2_, and it obtains the global optimum within 100000 function evaluations. On *f*_3_, all the methods have similar convergence trends, but IGWO has the highest search accuracy, followed by DLGWO. On *f*_4_, GWOCS, MGWO, and IGWO can exploit the search space more successfully than the DLGWO, whereas the DLGWO takes the fourth place. The convergence rate for *f*_5_ is similar for all the algorithms, and they converge fast during a few iterations, but then reveal stagnation behaviors. On *f*_6_ and *f*_7_, DLGWO exhibits the fastest convergence speed and the highest convergence accuracy. The same trend can be observed on *f*_8_. On *f*_9_ and *f*_11_, DLGWO and other GWO variants can all locate the global optimum. On *f*_10_, DLGWO exhibits slightly higher convergence rate compared with other optimizers. On *f*_12_ and *f*_13_, DLGWO and RWGWO are top 2 optimizers, and they can explore the search space with more efficiency when other methods reach stagnation prematurely. According to these results, the utilized DLS and Levy flight in the proposed DLGWO algorithm can generally improve its convergence performance.

The article "Dimensional Learning Strategy-Based Grey Wolf Optimizer for Solving the Global Optimization Problem" was published in 2022. Journal: Comput Intell Neurosci.

### 5.6. Comparison of the DLGWO with Other Metaheuristics

In this section, the performance of the DLGWO is examined with other well-established metaheuristics which can be generally divided into two categories: (1) recently developed algorithms, including TLBO [19], SSA [20], SCA [21], WOA [22], and BOA [23]; (2) high-performance algorithms, including LSHADE [57] (champion optimizer in the CEC 2014 test) and LSHADE-cnEpSin [58] (champion optimizer in the CEC 2017 test). The parameter settings for these algorithms are given in Table 10. The experimental conditions are the same as in the previous section: all algorithms are implemented over 30 independent runs with 40 search agents and the maximum number of function evaluations of 300000.

### 5.7. Algorithm Accuracy Analysis

Table 11 provides the comparison results on unimodal functions. For the unimodal functions (*f*_1_–*f*_7_), DLGWO attains the best rank for 4 functions, i.e., *f*_1_, *f*_2_, *f*_4_, and *f*_7_, and obtains the global optimum for *f*_1_ and *f*_2_. LSHADE achieves the best rank for 5 functions, one more than the DLGWO, and finds the global optimum for *f*_1_, *f*_2_, *f*_3_, and *f*_6_, two more than the DLGWO. LSHADE-cnEpSin achieves the best rank for 4 functions, the same as the DLGWO, but also achieves the global optimum for *f*_1_, *f*_2_, *f*_3_, and *f*_6_, two more than the DLGWO. On *f*_4_, DLGWO obtains the highest accuracy of 9.57*E* − 148, which is a great superiority to LSHADE and LSHADE-cnEpSin. LSHADE and LSHADE-cnEpSin overtake the other methods on *f*_5_ with apparently higher search accuracy, and DLGWO comes in the third place. Compared with the rest metaheuristics, i.e., TLBO, SSA, SCA, WOA, and BOA, DLGWO exhibits distinguished performance since its average rank is smaller than these algorithms. To sum up, the proposed DLGWO shows strong performance on unimodal functions, but its exploitation ability is worse than CEC 2014 champion algorithm LSHADE and CEC 2017 champion algorithm LSHADE-cnEpSin. In the final rank, LSHADE-cnEpSin and LSHADE are the top 2 optimizers, with DLGWO ranking third, followed by TLBO, WOA, BOA and SSA (tied for the sixth place), and SCA. With respect to the multimodal functions (*f*_8_–*f*_13_) shown in Table 12, WOA outperforms the other methods on *f*_8_ with the highest accuracy of −1.23*E* + 04, followed by the proposed DLGWO with an accuracy of −8.29*E* + 03. Among 8 algorithms, 5 algorithms can achieve the global optimum on *f*_9_, i.e., SCA, WOA, LSHADE, LSHADE-cnEpSin, and DLGWO. On *f*_10_, LSHADE-cnEpSin has the best result, but DLGWO also obtains competitive result with an accuracy of 4.64*E* − 15. The global optimum of *f*_11_ can be achieved by 6 methods, i.e., TLBO, SCA, WOA, LSHADE, LSHADE-cnEpSin, and DLGWO. TLBO takes the first place on *f*_12_ with the highest search precision of 2.45*E* − 24, followed by LSHADE-cnEpSin and DLGWO. On *f*_13_, SSA is the most efficient optimizer. According to the average rank and final rank of these algorithms on multimodal problems, DLGWO is inferior to CEC 2017 champion algorithm LSHADE-cnEpSin, but outperforms CEC 2014 champion algorithm LSHADE with slight advantage, and is superior to the other algorithms. Hence, the experimental results demonstrate the exploration capacity of the proposed DLGWO.

The article "Dimensional Learning Strategy-Based Grey Wolf Optimizer for Solving the Global Optimization Problem" was published in 2022. Journal: Comput Intell Neurosci.

Table 13 gives the statistical results on the fixed-dimension multimodal functions (*f*_14_–*f*_23_). According to the obtained results in Table 13, SSA, SCA, LSHADE-cnEpSin, and DLGWO obtain the highest accuracy on *f*_14_, but SSA has the smallest standard deviation. On *f*_15_, LSHADE-cnEpSin achieves the best result with the highest search accuracy of 2.11*E* − 07, followed by LSHADE and BOA, with DLGWO ranking fourth. On *f*_16_–*f*_19_, all algorithms can obtain or locate close to the global optimum (−1.0316 for *f*_16_, 0.398 for *f*_17_, 3.00 for *f*_18_, and −3.86 for *f*_19_), but they have different standard deviations, which indicate different performance stability of algorithms. TLBO attains the smallest standard deviations for *f*_16_, *f*_17_, and *f*_19_. On *f*_18_, LSHADE and LSHADE-cnEpSin have the most robust performance and achieve the smallest standard deviations. LSHADE obtains the best result on *f*_20_, while DLGWO also provides competitive result with an accuracy of −3.28*E* + 00. On *f*_21_, WOA and DLGWO are the best performed algorithms, both methods achieve the highest search precision of −1.01*E* + 01, but the standard deviation of WOA is slightly smaller. On *f*_22_ and *f*_23_, DLGWO exhibits a noticeable advantage in terms of search precision and stability. From the average rank and final rank of these methods, DLGWO is the best optimizer in solving the fixed-dimension multimodal functions, with LSHADE-cnEpSin and LSHADE ranking second and third, followed by WOA and TLBO (tied for the fourth place), SSA, BOA, and SCA. Moreover, from Table 13, it can also be observed that DLGWO exhibits larger standard deviation on *f*_16_–*f*_19_ compared with several non-GWO competitors. The unstable performance on these functions can be attributed to the defect in the original GWO design that has a search tendency towards the origin of the coordinate system. When the global optimum of functions is shifted from the origin, this defect can affect the GWO and its modified variants [59].

The article "Dimensional Learning Strategy-Based Grey Wolf Optimizer for Solving the Global Optimization Problem" was published in 2022. Journal: Comput Intell Neurosci.

Tables 14 and 15 provide the overall Wilcoxon rank-sum test results between DLGWO and each metaheuristic. From Table 14, DLGWO generally shows strong performance in comparison with other non-GWOs. Even compared with CEC 2017 champion algorithm LSHADE-cnEpSin and CEC 2014 champion algorithm LSHADE, DLGWO can obtain competitive results of 7/8/8 and 7/10/6, respectively. With regard to the rest optimizers, it shows superior performance and achieves results of 13/4/6 vs. TLBO, 15/1/7 vs. SSA, 19/4/0 vs. SCA, 12/7/4 vs. WOA, and 18/4/1 vs. BOA.

### 5.8. Convergence Behavior Analysis

The convergence curves of the DLGWO and the other metaheuristics based on 4 test functions are presented in Figure 11. As shown in Figure 11, DLGWO has the fastest convergence speed on *f*_2_, followed by LSHADE-cnEpSin and LSHADE. WOA does not converge fast in the initial stage of iterations, but it then accelerates and converges fast in further iterations. As for the other methods SSA, SCA, and BOA, they converge prematurely and cannot find solutions with high accuracy. On *f*_3_, LSHADE-cnEpSin and LSHADE have the highest convergence accuracy, although they cannot converge fast in the first half of iterations. DLGWO is inferior to these two algorithms in terms of search accuracy, but it shows an agreeable convergence behavior during the whole iterative course and has a strong ability to resist the trapping of local optima. By contrast, WOA, SSA, SCA, and BOA suffer from the immature stagnation. With regard to *f*_9_, DLGWO has the fastest convergence speed and achieves the global optimum at a very early stage of the iterations. On *f*_10_, the convergence accuracy of the DLGWO is slightly lower than that of LSHADE-cnEpSin and LSHADE, but DLGWO has the second fastest convergence rate, only inferior to TLBO. From the above analysis, DLGWO is effective with regard to convergence accuracy and speed compared with other metaheuristics.

The article "Dimensional Learning Strategy-Based Grey Wolf Optimizer for Solving the Global Optimization Problem" was published in 2022. Journal: Comput Intell Neurosci.

## 6. DLGWO for Real-World Optimization Problems

In this section, the proposed DLGWO is implemented on three classical engineering optimization problems, tension/compression spring design, welded beam design, and pressure vessel design, to verify its performance in solving real-world problems. These three problems are often employed as classical constrained optimization problems [60, 61]. For a fair comparison, the experiments on the DLGWO and the other optimizers mentioned above are conducted on the same platform based on 30 independent executions with 40 search agents and 100000 function evaluations.

### 6.1. Tension/Compression Spring Design

This is a well-known optimization problem. The structure of a tension/compression spring is shown in Figure 12. The objective is to find the minimum weight of a spring with constraints on shear stress, surge frequency, and minimum deflection. Three decision variables are involved in the problem: wire diameter (*d*), mean coil diameter (*D*), and active coil number (*N*).

The mathematical formulation of this problem is as follows:

(17) $$\begin{array}{c} \begin{array}{cc} \text{ Consider } & \left[x_{1},x_{2},x_{3}\right]=\left[d,D,N\right]\\ \text{ Minimize } & f\left(x\right)=x_{1}^{2}x_{2}\left(x_{3}+2\right)\\ \text{ subject to } & g_{1}\left(x\right)=1-\frac{x_{2}^{3}x_{3}}{71785x_{1}^{4}}\leq 0\\ g_{2}\left(x\right)=\frac{1}{5108x_{1}^{2}}+\frac{4x_{2}^{2}-x_{1}x_{2}}{12566\left(x_{1}^{3}x_{2}-x_{1}^{4}\right)}-1\leq 0\\ g_{3}\left(x\right)=1-\frac{140.45x_{1}}{x_{2}^{2}x_{3}}\leq 0\\ g_{4}\left(x\right)=\frac{x_{1}+x_{2}}{1.5}-1\leq 0\\ \text{ Range of variables: } & 0.05\leq x_{1}\leq 2\\ 0.25\leq x_{2}\leq 1.3\\ 2\leq x_{3}\leq 15 \end{array}. \end{array}$$

The numerical results obtained by the DLGWO are compared with other optimization algorithms such as GWO, learnGWO, GSA, SCA, MVO, HHO, and LSHADE, and the comparison results are listed in Table 16. As shown in Table 16, the minimum weight for the compression/tension spring is achieved by LSHADE. Although the DLGWO is inferior to LSHADE, it is the second best optimizer for the compression/tension spring problem with a promising optimization performance.

### 6.2. Welded Beam Design

The goal of this problem is to obtain the minimum cost of the welded beam subject to constraints including bending stress (*σ*), shear stress (*τ*), buckling load (*P*_*c*_), beam deflection (*δ*), and other side constraints. The four design variables related to the problem are weld thickness (*h*), length of the beam attached to the weld (*l*), height of the beam (*t*), and thickness of the beam (*b*). The schematic of this problem is illustrated in Figure 13.

The article "Dimensional Learning Strategy-Based Grey Wolf Optimizer for Solving the Global Optimization Problem" was published in 2022. Journal: Comput Intell Neurosci.

This problem can be mathematically expressed as follows:

(18) $$\begin{array}{c} \begin{array}{cc} \text{ Consider } & \left[y_{1},y_{2},y_{3},y_{4}\right]=\left[h,l,t,b\right]\\ \text{ Minimize } & f\left(y\right)=1.10471y_{1}^{2}y_{2}+0.0481y_{3}y_{4}\left(14.0+y_{2}\right)\\ \text{ subject to } & g_{1}\left(y\right)=\tau \left(y\right)-\tau_{\max}\leq 0\\ g_{2}\left(y\right)=\sigma \left(y\right)-\sigma_{\max}\leq 0\\ g_{3}\left(y\right)=y_{1}-y_{4}\leq 0\\ g_{4}\left(y\right)=\delta \left(y\right)-\delta_{\max}\leq 0\\ g_{5}\left(y\right)=P-P_{c}\left(y\right)\leq 0\\ g_{6}\left(y\right)=0.125-y_{1}\leq 0\\ g_{7}\left(y\right)=1.10471y_{1}^{2}+0.04811y_{3}y_{4}\left(14.0+y_{2}\right)-5.0\leq 0\\ \text{ Range of variables: } & 0.1\leq y_{1}\leq 2\\ 0.1\leq y_{2}\leq 10\\ 0.1\leq y_{3}\leq 10\\ 0.1\leq y_{4}\leq 2 \end{array}. \end{array}$$

Table 17 gives the numerical results obtained by the DLGWO and the other methods such as GWO, RWGWO, MFO, KH, BOA, SSA, MPA, and JADE. As demonstrated by Table 17, the minimum weight for the welded beam design problem is obtained by the DLGWO.

### 6.3. Pressure Vessel Design Problem

The pressure vessel design problem was proposed by Kannan and Kramer [68], and the goal of this problem is to obtain the minimum cost of a columnar vessel, which is shown in Figure 14.

The design variables are the thickness of the ball (*Th*), shell thickness (*Ts*), shell length (*l*), and inside radius (*R*). The mathematical model can be expressed as follows:

(19) $$\begin{array}{c} \begin{array}{cc} \text{ Consider } & \left[z_{1},z_{2},z_{3},z_{4}\right]=\left[T_{s},T_{h},R,l\right]\\ \text{ Minimize } & f\left(z\right)=0.6224z_{1}z_{3}z_{4}+1.7881z_{2}z_{3}^{2}+3.1661z_{1}^{2}z_{4}+19.84z_{1}^{2}z_{3}\\ \text{ subject to } & g_{1}\left(z\right)=-z_{1}+0.0193z_{3}\leq 0\\ g_{2}\left(z\right)=-z_{2}+0.00954z_{3}\leq 0\\ g_{3}\left(z\right)=-\pi z_{3}^{2}z_{4}-\frac{4}{3}\pi z_{3}^{3}+1296000\leq 0\\ g_{4}\left(z\right)=z_{4}-240\leq 0\\ \text{ Range of variables: } & 0\leq z_{1}\leq 100\\ 0\leq z_{2}\leq 100\\ 10\leq z_{3}\leq 200\\ 10\leq z_{4}\leq 200 \end{array}. \end{array}$$

The optimization results for the pressure vessel design problem are listed in Table 18. The compared algorithms are GWO, EEGWO, CMA-ES, TSO, CSA, EO, TLBO, and DA. From Table 18, DLGWO can provide an excellent parameter design plan with lower cost compared to other algorithms.

The article "Dimensional Learning Strategy-Based Grey Wolf Optimizer for Solving the Global Optimization Problem" was published in 2022. Journal: Comput Intell Neurosci.

## 7. Conclusion

This paper introduces DLS into the leading hierarchy of the GWO algorithm. During the process of the DLS, the delta wolf learns from the corresponding dimensions of both alpha and beta wolves to construct an exemplar wolf. Instead of learning from the three dominant wolves in each iteration, the search agents learn from the exemplar wolf which is composed of the excellent information learned from the three dominant wolves. This improves the efficiency of utilizing the population information of the GWO. Moreover, the Levy flight is adopted to reinforce the global exploration ability. Based on these two strategies, the DLGWO algorithm is proposed. To verify the validity of the proposed method for solving global optimization problems, DLGWO is compared with some variants of the GWO and some other metaheuristics based on 23 widely utilized benchmark functions. The experimental results of the benchmark functions manifest that the DLGWO exhibits a promising search performance and has a good balance between exploitation and exploration. Furthermore, DLGWO is implemented into three engineering problems, and the statistical results verify that the proposed DLGWO is an efficient and stable optimization method.

## Figures and Tables

**Figure 1:** Hunting behavior of grey wolves.

**Figure 2:** Conflicting guidance of the three dominant wolves.

**Figure 3:** Process of the DLS.

**Figure 4:** DLS flowchart.

**Figure 5:** 2D and 3D trajectories drawn from the Levy distribution.

**Figure 6:** DLGWO method.

**Figure 7:** Demonstration of benchmark functions.

**Figure 8:** Comparison of search history, trajectories, and diversity between solutions of the DLGWO, DLSGWO, and LFGWO.

**Figure 9:** Convergence behavior on test functions *f*_1_–*f*_4_.

**Figure 10:** Convergence behavior on test functions *f*_5_–*f*_13_.

**Figure 11:** Convergence behavior on test functions.

**Figure 12:** Tension-compression spring.

**Figure 13:** Welded beam design.

**Figure 14:** Pressure vessel design problem.

**Algorithm 1:** The pseudo-code of the standard GWO.

**Algorithm 2:** Constructing the exemplar *x*_*i*_^*dl*^.

**Algorithm 3:** Constructing the exemplar wolf according to the three dominant wolves.

**Table 1:** Benchmark functions.

Function name	Expression	Dim	Range	*f*_min_
Sphere	*f*_1_(*x*)=∑_*i*=1_^*D*^*xi*^2^	30	[−100,100]^*D*^	0
Schwefel's problem 2.22	*f*_2_(*x*)=∑_*i*=1_^*D*^|*x*_*i*_|+∏_*i*=1_^*D*^|*x*_*i*_|	30	[−10,10]^*D*^	0
Schwefel's problem 1.2	*f*_3_(*x*)=∑_*i*=1_^*D*^(∑_*j*=1_^*i*^*x*_*j*_)^2^	30	[−100,100]^*D*^	0
Schwefel's problem 2.21	$f_{4}\left(x\right)=\underset{i}{\text{max}}\left\{\left|x_{i}\right|,\;1\leq i\leq D\right\}$	30	[−100,100]^*D*^	0
Rosenbrock	*f*_5_(*x*)=∑_*i*=1_^*D*−1^(100(*x*_*i*+1_ − *x*_*i*_^2^)^2^+(*x*_*i*_ − 1)^2^)	30	[−30,30]^*D*^	0
Step	*f*_6_(*x*)=∑_*i*=1_^*D*^(⌊*x*_*i*_+0.5⌋^2^)	30	[−100,100]^*D*^	0
Noisy quartic	*f*_7_(*x*)=∑_*i*=1_^*D*^*ix*_*i*_^4^+random[0,1]	30	[−1.28, 1.28]^*D*^	0
Schwefel's problem 2.26	$f_{8}\left(x\right)=-\sum_{i=1}^{D}\left(x_{i}\sin\left(\sqrt{\left|x_{i}\right|}\right)\right)$	30	[−100,100]^*D*^	−12569.5
Rastrigin	*f*_9_(*x*)=∑_*i*=1_^*D*^[*x*_*i*_^2^ − 10*cos*(2*πx*_*i*_)+10]	30	[−5.12, 5.12]^*D*^	0
Ackley	$f_{10}\left(x\right)=-20\;\exp\left(-0.2\sqrt{1/D\sum_{i=1}^{D}x_{i}^{2}}\right)-\exp\left(1/D\sum_{i=1}^{D}\cos\left(2\pi x_{i}\right)\right)+20+e$	30	[−32,32]^*D*^	0
Griewank	$f_{11}\left(x\right)=1/4000\sum_{i=1}^{D}x_{i}^{2}-\prod_{i=1}^{D}\cos\left(x_{i}/\sqrt{i}\right)+1$	30	[−600,600]^*D*^	0
Penalized 1	$\begin{array}{cc} f_{12}\left(x\right)= & \pi /D\left\{\sum_{i=1}^{D-1}\left[1+10\;\sin^{2}\left(\pi y_{i+1}\right)\right]+{\left(y_{N}-1\right)}^{2}+\right.\\ \left.\left(10\;\sin^{2}\left(\pi y_{1}\right)\right)\right\}+\sum_{i=1}^{D}u\left(x_{i},10,100,4\right)\\ y_{i}=1+x_{i}+1/4\\ u\left(x_{i},a,k,m\right)=\left\{\begin{array}{cc} k{\left(x_{i}-a\right)}^{m}, & x_{i}\rangle a\\ 0, & -a\leq x_{i}\leq a\\ k{\left(-x_{i}-a\right)}^{m}, & x_{i}\langle -a \end{array}\right. \end{array}$	30	[−50,50]^*D*^	0
Penalized 2	$\begin{array}{cc} f_{13}\left(x\right)= & 0.1\left\{\sin^{2}\left(3\pi x_{1}\right)+\sum_{i=1}^{D-1}{\left(x_{i}-1\right)}^{2}\left[1+\;\sin^{2}\left(3\pi x_{i+1}\right)\right]+\right.\\ \left.{\left(x_{D}-1\right)}^{2}\left[1+\;\sin^{2}\left(2\pi x_{D}\right)\right]\right\}+\sum_{i=1}^{D}u\left(x_{i},5,100,4\right) \end{array}$	30	[−50,50]^*D*^	0
Shekel's Foxholes function	*f*_14_(*x*)=(1/500+∑_*j*=1_^25^1/*j*+∑_*i*=1_^2^(*x*_*i*_ − *a*_*i*,*j*_)^6^)^−1^	2	[−65,65]^*D*^	0.998
Kowalik's function	*f*_15_(*x*)=∑_*i*=1_^11^[*a*_*i*_ − ((*x*_1_(*b*_*i*_^2^+*b*_*i*_*x*_2_))/(*b*_*i*_^2^+*b*_*i*_*x*_3_+*x*_4_))]^2^	4	[−5,5]^*D*^	0.003
Six-hump camel back	$f_{16}\left(x\right)=4x_{1}^{2}-2.1x_{1}^{4}+\frac{1}{3}x_{1}^{6}+x_{1}x_{2}-4x_{2}^{2}+4x_{2}^{4}$	2	[−5,5]^*D*^	−1.0316
Branin	*f*_17_(*x*)=(*x*_2_ − 5.1/4*π*^2^*x*_1_^2^+5/*πx*_1_ − 6)^2^+10(1 − 1/8*π*)cos *x*_1_+10	2	[−5,5]^*D*^	0.398
Goldstein–Price function	*f*_18_(*x*)=[1+(*x*_1_+*x*_2_+1)^2^(19 − 14*x*_1_+3*x*_1_^2^ − 14*x*_2_+6*x*_1_*x*_2_+3*x*_2_^2^)]	2	[−2,2]^*D*^	3.00
	×[30+(2*x*_1_ − 3*x*_2_)^2^ × (18 − 32*x*_1_+12*x*_1_^2^+48*x*_2_ − 36*x*_1_*x*_2_+27*x*_2_^2^)]			
Hartmann 1	*f*_19_(*x*)=−∑_*i*=1_^4^*c*_*i*_exp[−∑_*j*=1_^3^*a*_*ij*_(*x*_*j*_ − *p*_*ij*_)^2^]	3	[1,3]^*D*^	−3.86
Hartmann 2	*f*_20_(*x*)=−∑_*i*=1_^4^*c*_*i*_exp[−∑_*j*=1_^6^*a*_*ij*_(*x*_*j*_ − *p*_*ij*_)^2^]	6	[0,1]^*D*^	−3.32
Shekel 1	*f*_21_(*x*)=−∑_*i*=1_^5^[(*X* − *a*_*i*_)(*X* − *a*_*i*_)^*T*^+*c*_*i*_]^−1^	4	[−10,10]^*D*^	−10.1532
Shekel 2	*f*_22_(*x*)=−∑_*i*=1_^7^[(*X* − *a*_*i*_)(*X* − *a*_*i*_)^*T*^+*c*_*i*_]^−1^	4	[−10,10]^*D*^	−10.4028
Shekel 3	*f*_23_(*x*)=−∑_*i*=1_^10^[(*X* − *a*_*i*_)(*X* − *a*_*i*_)^*T*^+*c*_*i*_]^−1^	4	[−10,10]^*D*^	−10.5363

The article "Dimensional Learning Strategy-Based Grey Wolf Optimizer for Solving the Global Optimization Problem" was published in 2022. Journal: Comput Intell Neurosci.

**Table 2:** Comparison results for the DLGWO, LFGWO, and DLSGWO.

	Metrics	DLSGWO	LFGWO	DLGWO
*f*_1_	Mean	0.00*E* + 00	9.25*E* − 273	0.00*E* + 00
	SD	0.00*E* + 00	1.51*E* − 272	0.00*E* + 00
	Rank	1	3	1

*f*_2_	Mean	0.00*E* + 00	1.13*E* − 282	0.00*E* + 00
	SD	0.00*E* + 00	8.46*E* − 282	0.00*E* + 00
	Rank	1	3	1

*f*_3_	Mean	6.03*E* − 192	8.19*E* − 28	6.27*E* − 182
	SD	7.68*E* − 191	1.60*E* − 27	1.01*E* − 182
	Rank	1	3	2

*f*_4_	Mean	7.11*E* − 188	1.33*E* − 115	9.07*E* − 150
	SD	1.58*E* − 189	1.06*E* − 116	1.26*E* − 151
	Rank	1	3	2

*f*_5_	Mean	2.47*E* + 01	2.71*E* + 01	2.35*E* + 01
	SD	1.23*E* + 00	1.04*E* + 00	3.08*E* − 01
	Rank	2	3	1

*f*_6_	Mean	1.24*E* − 06	1.86*E* − 01	1.08*E* − 06
	SD	3.61*E* − 07	1.06*E* − 01	3.93*E* − 07
	Rank	2	3	1

*f*_7_	Mean	1.01*E* − 05	6.12*E* − 04	1.44*E* − 05
	SD	8.51*E* − 06	2.73*E* − 04	5.18*E* − 05
	Rank	1	3	2

Average rank for *f*_1_–*f*_7_		1.28	3.00	1.42

*f*_8_	Mean	−7.21*E* + 03	−7.92*E* + 03	−8.33*E* + 03
	SD	1.07*E* + 03	5.46*E* + 02	2.25*E* + 02
	Rank	3	2	1

*f*_9_	Mean	0.00*E* + 00	0.00*E* + 00	0.00*E* + 00
	SD	0.00*E* + 00	0.00*E* + 00	0.00*E* + 00
	Rank	1	1	1

*f*_10_	Mean	8.97*E* − 15	4.44*E* − 15	4.95*E* − 15
	SD	8.89*E* − 15	1.58*E* − 15	3.17*E* − 15
	Rank	3	1	2

*f*_11_	Mean	1.25*E* − 03	0.00*E* + 00	0.00*E* + 00
	SD	2.81*E* − 03	0.00*E* + 00	0.00*E* + 00
	Rank	3	1	1

*f*_12_	Mean	6.54*E* − 03	1.74*E* − 08	1.68*E* − 08
	SD	4.62*E* − 03	5.73*E* − 09	9.08*E* − 09
	Rank	3	2	1

*f*_13_	Mean	3.09*E* − 05	9.63*E* − 06	2.88*E* − 07
	SD	1.31*E* − 06	7.04*E* − 07	1.82*E* − 07
	Rank	3	2	1

Average rank for *f*_8_–*f*_13_		2.66	1.50	1.16

Average rank for *f*_1_–*f*_13_		1.92	2.30	1.31

**Table 3:** Comparison results on benchmark functions with different dimensions.

	Dim	10		30		100		200	
	Metrics	GWO	DLGWO	GWO	DLGWO	GWO	DLGWO	GWO	DLGWO
*f*_1_	Mean	**0.00*E* + 00**	**0.00*E* + 00**	**0.00*E* + 00**	**0.00*E* + 00**	3.92*E* − 262	**2.48*E* − 286**	2.95*E* − 129	**1.67*E* − 162**
	SD	0.00*E* + 00	0.00*E* + 00	0.00*E* + 00	0.00*E* + 00	5.88*E* − 263	0.00*E* + 00	6.44*E* − 128	9.88*E* − 163

*f*_2_	Mean	**0.00*E* + 00**	**0.00*E* + 00**	**0.00*E* + 00**	**0.00*E* + 00**	**0.00*E* + 00**	**0.00*E* + 00**	2.23*E* − 218	**8.43*E* − 237**
	SD	0.00*E* + 00	0.00*E* + 00	0.00*E* + 00	0.00*E* + 00	0.00*E* + 00	0.00*E* + 00	7.05*E* − 217	5.75*E* − 237

*f*_3_	Mean	5.69*E* − 188	**3.86*E* − 230**	1.05*E* − 156	**6.10*E* − 184**	5.61*E* − 105	**1.52*E* − 110**	**1.94*E* + 00**	3.16*E* + 00
	SD	2.76*E* − 187	8.22*E* − 231	9.01*E* − 157	5.41*E* − 184	9.65*E* − 105	7.52*E* − 111	8.08*E* − 01	1.22*E* + *E* + 00

*f*_4_	Mean	1.09*E* − 293	**1.33*E* − 322**	5.45*E* − 121	**9.36*E* − 150**	3.16*E* − 26	**2.79*E* − 38**	3.91*E* − 01	**1.99*E* − 03**
	SD	2.24*E* − 294	3.69*E* − 323	6.56*E* − 121	2.51*E* − 151	2.35*E* − 26	6.75*E* − 38	1.52*E* − 01	1.47*E* − 03

*f*_5_	Mean	6.22*E* + 00	**2.76*E* + 00**	2.77*E* + 01	**2.36*E* + 01**	9.61*E* + 01	**9.41*E* + 01**	**1.92*E* + 02**	1.98*E* + 02
	SD	2.62*E* − 01	7.84*E* − 01	9.34*E* − 01	4.22*E* − 01	3.16*E* − 01	5.02*E* − 01	2.38*E* − 01	1.09*E* − 01

*f*_6_	Mean	7.06*E* − 01	**2.53*E* − 08**	5.96*E* − 01	**4.55*E* − 07**	1.49*E* + 00	**2.50*E* − 03**	2.74*E* + 00	**7.29*E* − 01**
	SD	5.26*E* − 02	3.12*E* − 08	3.45*E* − 01	2.46*E* − 07	7.94*E* − 01	2.41*E* − 04	1.74*E* + 00	2.24*E* − 01

*f*_7_	Mean	9.55*E* − 05	**2.27*E* − 05**	4.28*E* − 05	**1.09*E* − 05**	8.26*E* − 03	**6.04*E* − 04**	1.44*E* − 02	**2.56*E* − 04**
	SD	5.79*E* − 04	1.37*E* − 05	3.07*E* − 05	8.99*E* − 06	3.22*E* − 04	9.90*E* − 05	8.88*E* − 03	2.11*E* − 04

*f*_8_	Mean	−3.40*E* + 03	**−4.35*E* + 03**	−6.57*E* + 03	**−8.29*E* + 03**	−1.61*E* + 04	**−2.02*E* + 04**	−2.85*E* + 04	**−3.48*E* + 04**
	SD	2.34*E* + 02	5.75*E* + 01	5.25*E* + 02	8.77*E* + 02	4.31*E* + 02	1.74*E* + 02	5.54*E* + 04	6.39*E* + 02

*f*_9_	Mean	**0.00*E* + 00**	**0.00*E* + 00**	**0.00*E* + 00**	**0.00*E* + 00**	**0.00*E* + 00**	**0.00*E* + 00**	1.14*E* − 13	**0.00*E* + 00**
	SD	0.00*E* + 00	0.00*E* + 00	0.00*E* + 00	0.00*E* + 00	0.00*E* + 00	0.00*E* + 00	8.84*E* − 14	0.00*E* + 00

*f*_10_	Mean	7.99*E* − 15	**4.44*E* − 15**	9.02*E* − 15	**4.84*E* − 15**	2.22*E* − 14	**1.51*E* − 14**	2.93*E* − 14	**2.22*E* − 14**
	SD	2.15*E* − 15	1.17*E* − 15	1.73*E* − 15	1.34*E* − 15	5.31*E* − 15	3.33*E* − 15	7.63*E* − 14	4.75*E* − 15

*f*_11_	Mean	**0.00*E* + 00**	**0.00*E* + 00**	**0.00*E* + 00**	**0.00*E* + 00**	**0.00*E* + 00**	**0.00*E* + 00**	**0.00*E* + 00**	**0.00*E* + 00**
	SD	0.00*E* + 00	0.00*E* + 00	0.00*E* + 00	0.00*E* + 00	0.00*E* + 00	0.00*E* + 00	0.00*E* + 00	0.00*E* + 00

*f*_12_	Mean	1.01*E* − 01	**5.48*E* − 08**	2.74*E* − 02	**1.72*E* − 08**	2.18*E* − 01	**8.26*E* − 04**	4.12*E* − 01	**3.92*E* − 03**
	SD	1.82*E* − 02	1.04*E* − 09	8.62*E* − 03	4.69*E* − 09	3.44*E* − 01	1.36*E* − 03	4.17*E* − 01	8.10*E* − 02

*f*_13_	Mean	9.67*E* − 01	**4.96*E* − 08**	7.02*E* − 01	**2.38*E* − 07**	4.72*E* + 00	**4.34*E* − 01**	**1.51*E* + 01**	2.06*E* + 01
	SD	2.01*E* − 01	5.90*E* − 08	2.18*E* − 01	5.91*E* − 08	2.16*E* + 01	9.59*E* − 01	8.10*E* + 00	6.55*E* + 00

The article "Dimensional Learning Strategy-Based Grey Wolf Optimizer for Solving the Global Optimization Problem" was published in 2022. Journal: Comput Intell Neurosci.

**Table 4:** Parameter settings and explanations for all versions of the GWO.

Name	Explanation	Parameters
GWO		*a* = [2,0]
RWGWO [39]	GWO with random walk	*a* = [2,0]
learnGWO [50]	GWO with improved hierarchy	*a* = [2,0], *θ*_*α*_ = 0.004715, *θ*_*β*_ = *θ*_*δ*_ = 0.00647
GWOCS [44]	GWO hybridized with cuckoo search	*a* = [2,0]
IGWO [56]	GWO with individual memory	*a* = [2,0], *b*_1_ = 0.6, *b*_2_ = 0.4, *p* = 0.5
SOGWO [43]	GWO with opposition-based learning	*a* = [2,0]
MGWO [34]	GWO with modified parameter *C*	*a* = [2,0]

**Table 5:** Results on benchmark functions *f*_1_–*f*_7_.

	Metrics	GWO	RWGWO	learnGWO	GWOCS	IGWO	SOGWO	MGWO	DLGWO
*f*_1_	Mean	0.00*E* + 00	0.00*E* + 00	0.00*E* + 00	0.00*E* + 00	0.00*E* + 00	0.00*E* + 00	0.00*E* + 00	0.00*E* + 00
	SD	0.00*E* + 00	0.00*E* + 00	0.00*E* + 00	0.00*E* + 00	0.00*E* + 00	0.00*E* + 00	0.00*E* + 00	0.00*E* + 00
	Rank	1	1	1	1	1	1	1	1

*f*_2_	Mean	1.80*E* − 284	5.40*E* − 223	4.98*E* − 291	0.00*E* + 00	0.00*E* + 00	1.33*E* − 287	0.00*E* + 00	0.00*E* + 00
	SD	1.07*E* − 284	0.00*E* + 00	0.00*E* + 00	0.00*E* + 00	0.00*E* + 00	4.90*E* − 290	0.00*E* + 00	0.00*E* + 00
	Rank	7	8	5	1	1	6	1	1

*f*_3_	Mean	6.82*E* − 151	1.30*E* − 153	1.80*E* − 162	4.98*E* − 180	8.42*E* − 192	5.40*E* − 153	2.10*E* − 176	6.53*E* − 182
	SD	2.32*E* − 152	1.66*E* − 153	6.06*E* − 161	2.49*E* − 180	7.62*E* − 191	2.67*E* − 153	5.27*E* − 175	3.34*E* − 182
	Rank	8	7	5	3	1	6	4	2

*f*_4_	Mean	5.45*E* − 121	7.53*E* − 116	6.72*E* − 126	7.23*E* − 213	7.54*E* − 155	1.83*E* − 122	5.38*E* − 190	9.36*E* − 150
	SD	6.56*E* − 121	2.86*E* − 117	1.78*E* − 127	0.00*E* + 00	4.83*E* − 155	8.25*E* − 123	3.85*E* − 191	2.51*E* − 151
	Rank	7	8	5	1	3	6	2	4

*f*_5_	Mean	2.73*E* + 01	2.66*E* + 01	2.63*E* + 01	2.64*E* + 01	2.61*E* + 01	2.49*E* + 01	2.77*E* + 01	2.33*E* + 01
	SD	9.47*E* − 01	4.96*E* − 01	3.61*E* − 01	8.39*E* − 01	7.79*E* − 01	7.26*E* − 02	7.53*E* − 01	4.19*E* − 01
	Rank	7	6	4	5	3	2	8	1

*f*_6_	Mean	6.06*E* − 01	1.88*E* − 07	6.01*E* − 01	1.21*E* + 00	9.59*E* − 02	9.98*E* − 01	1.60*E* + 00	4.28*E* − 07
	SD	3.78*E* − 01	3.88*E* − 08	2.43*E* − 01	3.63*E* − 01	2.18*E* − 02	9.64*E* − 02	4.31*E* − 02	1.06*E* − 07
	Rank	5	1	4	7	3	6	8	2

*f*_7_	Mean	5.18*E* − 05	3.76*E* − 04	5.16*E* − 04	6.97*E* − 05	1.93*E* − 05	7.73*E* − 05	4.22*E* − 05	1.21*E* − 05
	SD	2.68*E* − 05	4.27*E* − 05	1.39*E* − 05	3.31*E* − 05	9.21*E* − 04	2.93*E* − 05	2.05*E* − 05	8.99*E* − 05
	Rank	4	7	8	5	2	6	3	1

Average rank for *f*_1_ − *f*_7_		5.57	5.42	4.57	3.28	2.00	4.71	3.85	1.71

Final rank for *f*_1_ − *f*_7_		8	7	5	3	2	6	4	1

**Table 6:** Results on benchmark functions *f*_8_–*f*_13_.

	Metrics	GWO	RWGWO	learnGWO	GWOCS	IGWO	SOGWO	MGWO	DLGWO
*f*_8_	Mean	−5.99*E* + 03	−7.53*E* + 03	−5.27*E* + 03	−4.81*E* + 03	−7.29*E* + 03	−4.94*E* + 03	−6.51*E* + 03	−8.35*E* + 03
	SD	1.16*E* + 02	4.83*E* + 02	1.25*E* + 03	1.54*E* + 03	4.27*E* + 02	1.12*E* + 03	5.33*E* + 02	8.65*E* + 02
	Rank	5	2	6	8	3	7	4	1

*f*_9_	Mean	0.00*E* + 00	0.00*E* + 00	0.00*E* + 00	0.00*E* + 00	0.00*E* + 00	0.00*E* + 00	0.00*E* + 00	0.00*E* + 00
	SD	0.00*E* + 00	0.00*E* + 00	0.00*E* + 00	0.00*E* + 00	0.00*E* + 00	0.00*E* + 00	0.00*E* + 00	0.00*E* + 00
	Rank	1	1	1	1	1	1	1	1

*f*_10_	Mean	8.97*E* − 15	7.99*E* − 15	7.99*E* − 15	7.99*E* − 15	4.44*E* − 15	8.22*E* − 15	8.05*E* − 15	4.94*E* − 15
	SD	1.73*E* − 15	0.00*E* + 00	0.00*E* + 00	0.00*E* + 00	0.00*E* + 00	1.34*E* − 15	4.42*E* − 16	1.34*E* − 15
	Rank	8	3	3	3	1	7	6	2

*f*_11_	Mean	0.00*E* + 00	0.00*E* + 00	0.00*E* + 00	0.00*E* + 00	0.00*E* + 00	0.00*E* + 00	0.00*E* + 00	0.00*E* + 00
	SD	0.00*E* + 00	0.00*E* + 00	0.00*E* + 00	0.00*E* + 00	0.00*E* + 00	0.00*E* + 00	0.00*E* + 00	0.00*E* + 00
	Rank	1	1	1	1	1	1	1	1

*f*_12_	Mean	2.76*E* − 02	4.70*E* − 05	4.57*E* − 02	6.67*E* − 02	3.46*E* − 02	2.07*E* − 02	1.12*E* − 01	1.75*E* − 08
	SD	8.68*E* − 03	1.13*E* − 04	2.35*E* − 02	2.27*E* − 02	1.29*E* − 02	6.17*E* − 09	5.33*E* − 02	4.70*E* − 09
	Rank	5	2	3	6	8	4	7	1

*f*_13_	Mean	7.48*E* − 01	3.57*E* − 07	5.27*E* − 01	6.66*E* − 01	5.76*E* − 01	3.08*E* − 07	7.21*E* − 01	2.42*E* − 07
	SD	2.38*E* − 01	5.29*E* − 08	2.67*E* − 01	1.99*E* − 01	2.06*E* − 01	6.80*E* − 08	2.68*E* − 01	6.31*E* − 08
	Rank	8	2	5	6	4	3	7	1

Average rank for *f*_8_ − *f*_13_		4.67	1.83	3.17	4.17	3.00	3.83	4.33	1.17

Final rank for *f*_8_ − *f*_13_		8	2	4	6	3	5	7	1

The article "Dimensional Learning Strategy-Based Grey Wolf Optimizer for Solving the Global Optimization Problem" was published in 2022. Journal: Comput Intell Neurosci.

**Table 7:** Results on benchmark functions *f*_14_–*f*_23_.

	Metrics	GWO	RWGWO	learnGWO	GWOCS	IGWO	SOGWO	MGWO	DLGWO
*f*_14_	Mean	4.92*E* + 00	9.98*E* − 01	7.41*E* + 00	4.35*E* + 00	6.29*E* + 00	9.98*E* − 01	8.81*E* + 00	9.98*E* − 01
	SD	4.05*E* + 00	8.27*E* − 14	4.86*E* + 00	4.46*E* + 00	5.46*E* + 00	3.83*E* − 13	4.04*E* + 00	3.83*E* − 13
	Rank	5	1	7	4	6	2	8	2

*f*_15_	Mean	6.03*E* − 03	6.69*E* − 04	3.17*E* − 03	3.08*E* − 04	3.43*E* − 03	3.10*E* − 04	4.38*E* − 04	3.07*E* − 04
	SD	9.78*E* − 03	4.57*E* − 04	7.58*E* − 03	4.86*E* − 07	7.47*E* − 03	1.73*E* − 08	3.46*E* − 04	3.33*E* − 10
	Rank	8	5	6	2	7	3	4	1

*f*_16_	Mean	−1.03*E* + 00	−1.03*E* + 00	−1.03*E* + 00	−1.03*E* + 00	−1.03*E* + 00	−1.03*E* + 00	−1.03*E* + 00	−1.03*E* + 00
	SD	7.66*E* − 11	4.59*E* − 11	5.77*E* − 11	1.79*E* − 07	6.64*E* − 10	7.49*E* − 11	6.30*E* − 11	1.03*E* − 11
	Rank	6	2	3	8	7	5	4	1

*f*_17_	Mean	3.97*E* − 01	3.97*E* − 01	3.97*E* − 01	3.97*E* − 01	3.97*E* − 01	3.97*E* − 01	3.97*E* − 01	3.97*E* − 01
	SD	2.24*E* − 09	2.62*E* − 10	7.88*E* − 10	9.84*E* − 06	3.77*E* − 08	2.05*E* − 09	4.86*E* − 10	8.44*E* − 10
	Rank	6	1	3	8	7	5	2	4

*f*_18_	Mean	3.00*E* + 00	3.00*E* + 00	3.00*E* + 00	3.00*E* + 00	3.00*E* + 00	3.00*E* + 00	3.00*E* + 00	3.00*E* + 00
	SD	7.73*E* − 07	9.59*E* − 08	5.36*E* − 08	1.74*E* − 07	7.55*E* − 08	2.09*E* − 09	4.91*E* − 08	5.68*E* − 10
	Rank	8	6	4	7	5	2	3	1

*f*_19_	Mean	−3.86*E* + 00	−3.86*E* + 00	−3.86*E* + 00	−3.86*E* + 00	−3.86*E* + 00	−3.86*E* + 00	−3.86*E* + 00	−3.86*E* + 00
	SD	2.49*E* − 07	7.67*E* − 05	1.94*E* − 07	3.18*E* − 07	3.04*E* + 07	1.31*E* − 08	1.32*E* − 07	9.86*E* − 08
	Rank	5	8	4	7	6	1	3	2

*f*_20_	Mean	−3.24*E* + 00	−3.27*E* + 00	−3.24*E* + 00	−3.27*E* + 00	−3.26*E* + 00	−3.32*E* + 00	−3.18*E* + 00	−3.28*E* + 00
	SD	9.84*E* − 02	6.46*E* − 02	8.99*E* − 02	5.81*E* − 02	7.91*E* − 02	2.41*E* − 08	1.73*E* − 01	5.80*E* − 02
	Rank	7	4	6	3	5	1	8	2

*f*_21_	Mean	−8.72*E* + 00	−1.01*E* + 01	−8.69*E* + 00	−6.91*E* + 00	−9.42*E* + 00	−1.01*E* + 01	−9.42*E* + 00	−1.01*E* + 01
	SD	2.43*E* − 02	3.81*E* − 07	2.48*E* + 00	2.34*E* + 00	1.92*E* + 00	2.39*E* − 06	1.92*E* + 00	6.35*E* − 07
	Rank	6	1	7	8	4	3	4	2

*f*_22_	Mean	−9.89*E* + 00	−1.04*E* + 01	−9.87*E* + 00	−9.91*E* + 00	−9.92*E* + 01	−1.04*E* + 01	−1.04*E* + 01	−1.04*E* + 01
	SD	1.94*E* + 00	6.43*E* − 07	1.61*E* + 00	2.20*E* + 00	1.58*E* + 00	2.51*E* − 06	5.14*E* − 07	1.59*E* − 06
	Rank	7	2	8	6	5	4	1	3

*f*_23_	Mean	−9.95*E* + 00	−1.01*E* + 01	−9.40*E* + 00	−8.45*E* + 00	−1.01*E* + 01	−1.05*E* + 01	−9.76*E* + 00	−1.05*E* + 01
	SD	8.75*E* − 07	4.69*E* − 06	1.33*E* − 06	2.29*E* + 00	2.45*E* − 05	2.28*E* − 06	2.04*E* + 00	5.04*E* − 07
	Rank	5	3	7	8	4	2	6	1

Average rank for *f*_14_ − *f*_23_		6.30	3.30	5.50	6.10	5.60	2.80	4.30	1.90

Final rank for *f*_14_ − *f*_23_		8	3	5	7	6	2	4	1

The article "Dimensional Learning Strategy-Based Grey Wolf Optimizer for Solving the Global Optimization Problem" was published in 2022. Journal: Comput Intell Neurosci.

**Table 8:** Wilcoxon rank-sum test on benchmark functions.

DLGWO vs.	GWO		RWGWO		learnGWO		GWOCS		IGWO		SOGWO		MGWO	
	*p*		*p*		*p*		*p*		*p*		*p*		*p*	
*f*_1_	NaN	≈	NaN	≈	NaN	≈	NaN	≈	NaN	≈	NaN	≈	NaN	≈
*f*_2_	1.21*E* − 12	+	1.21*E* − 12	+	1.21*E* − 12	+	NaN	≈	NaN	≈	1.21*E* − 12	+	NaN	≈
*f*_3_	3.02*E* − 11	+	3.02*E* − 11	+	3.02*E* − 11	+	7.77*E* − 09	+	2.22*E* − 08	−	3.02*E* − 11	+	7.77*E* − 09	+
*f*_4_	1.21*E* − 12	+	1.21*E* − 12	+	1.21*E* − 12	+	1.21*E* − 12	−	3.20*E* − 10	−	1.21*E* − 12	+	3.02*E* − 11	−
*f*_5_	3.02*E* − 11	+	3.02*E* − 11	+	3.02*E* − 11	+	3.02*E* − 11	+	3.02*E* − 11	+	3.02*E* − 11	+	3.02*E* − 11	+
*f*_6_	3.02*E* − 11	+	5.09*E* − 06	−	3.02*E* − 11	+	3.02*E* − 11	+	3.02*E* − 11	+	3.02*E* − 11	+	3.02*E* − 11	+
*f*_7_	2.95*E* − 06	+	3.02*E* − 11	+	3.02*E* − 11	+	7.04*E* − 07	+	2.91*E* − 01	≈	5.12*E* − 10	+	2.78*E* − 03	+
*f*_8_	3.02*E* − 11	+	3.02*E* − 11	+	3.02*E* − 11	+	3.02*E* − 11	+	3.02*E* − 11	+	3.02*E* − 11	+	3.02*E* − 11	+
*f*_9_	NaN	≈	NaN	≈	NaN	≈	NaN	≈	NaN	≈	NaN	≈	NaN	≈
*f*_10_	4.50*E* − 11	+	3.24*E* − 07	+	3.24*E* − 07	+	3.24*E* − 07	+	4.72*E* − 08	−	4.12*E* − 06	+	5.27*E* − 06	+
*f*_11_	NaN	≈	NaN	≈	NaN	≈	NaN	≈	NaN	≈	NaN	≈	NaN	≈
*f*_12_	1.21*E* − 12	+	1.09*E* − 10	+	1.21*E* − 12	+	1.21*E* − 12	+	1.21*E* − 12	+	1.21*E* − 12	+	1.21*E* − 12	+
*f*_13_	1.21*E* − 12	+	6.54*E* − 09	+	1.21*E* − 12	+	1.21*E* − 12	+	1.21*E* − 12	+	2.12*E* − 09	+	1.21*E* − 12	+
*f*_14_	2.09*E* − 09	+	2.82*E* − 06	−	1.99*E* − 11	+	5.12*E* − 09	+	1.99*E* − 11	+	NaN	≈	1.99*E* − 11	+
*f*_15_	4.05*E* − 09	+	8.31*E* − 08	+	4.82*E* − 08	+	5.24*E* − 06	+	3.14*E* − 09	+	1.66*E* − 06	+	2.83*E* − 07	+
*f*_16_	3.22*E* − 06	+	1.92*E* − 04	+	1.49*E* − 05	+	1.05*E* − 08	+	2.31*E* − 08	+	6.91*E* − 06	+	8.05*E* − 06	+
*f*_17_	2.11*E* − 04	+	5.06*E* − 06	−	4.32*E* − 01	≈	4.05*E* − 11	+	6.43*E* − 09	+	2.84*E* − 04	+	4.22*E* − 04	−
*f*_18_	3.31*E* − 09	+	2.02*E* − 06	+	8.52*E* − 05	+	1.41*E* − 09	+	5.73*E* − 05	+	3.88*E* − 03	+	1.46*E* − 05	+
*f*_19_	4.33*E* − 05	+	2.39*E* − 11	+	7.15*E* − 05	+	9.18*E* − 10	+	2.00*E* − 05	+	1.10*E* − 05	−	8.62*E* − 05	+
*f*_20_	2.17*E* − 04	+	4.11*E* − 03	+	5.51*E* − 04	+	5.82*E* − 03	+	7.03*E* − 04	+	6.43*E* − 11	−	2.03*E* − 04	+
*f*_21_	6.55*E* − 05	+	1.89*E* − 02	≈	4.37*E* − 05	+	1.22*E* − 05	+	6.40*E* − 04	+	4.40*E* − 02	≈	8.17*E* − 04	+
*f*_22_	6.44*E* − 12	+	8.74*E* − 01	≈	6.44*E* − 12	+	6.44*E* − 12	+	6.44*E* − 12	+	8.99*E* − 01	≈	3.04*E* − 02	≈
*f*_23_	8.24*E* − 06	+	4.52*E* − 01	≈	1.52*E* − 06	+	2.33*E* − 08	+	2.31*E* − 01	≈	7.09*E* − 01		6.03*E* − 06	+

The article "Dimensional Learning Strategy-Based Grey Wolf Optimizer for Solving the Global Optimization Problem" was published in 2022. Journal: Comput Intell Neurosci.

**Table 9:** Statistical results of the Wilcoxon rank-sum test.

DLGWO vs.		*f*_1_–*f*_7_	*f*_8_–*f*_13_	*f*_14_–*f*_23_	Sum
Wilcoxon's rank-sum test (+/≈/−)	GWO	6/1/0	4/2/0	10/0/0	20/3/0
	RWGWO	5/1/1	4/2/0	5/3/2	14/6/3
	learnGWO	6/1/0	4/2/0	9/1/0	19/4/0
	GWOCS	4/2/1	4/2/0	10/0/0	18/4/1
	IGWO	2/3/2	3/2/1	9/1/0	14/6/3
	SOGWO	6/1/0	4/2/0	8/1/1	18/4/1
	MGWO	4/2/1	4/2/0	8/1/1	16/5/2

**Table 10:** Parameter settings of the tested algorithm.

Algorithms	Parameters
TLBO [19]	*TF* is randomly selected with 1 or 2
SSA [20]	*c*_1_ = [2,0]
SCA [21]	*a* = 2, *r*1 = [a,0]
WOA [22]	*a*_1_ = [2,0], *a*_2_ = [−1, −2]
BOA [23]	*p* = 0.6, *a* = 0.1, *c* = 0.01
LSHADE [57]	*p* = 0.11, *r*^*arc*^ = 2.6, *H* = 6
LSHADE-cnEpSin [58]	*P*_*b*_=0.4, *P*_*s*_=0.5, *p* = 0.11,
	*r* ^*arc*^ = 1.4, freq-inti = 0.5, *H* = 5

**Table 11:** Results on benchmark functions *f*_1_–*f*_7_.

	Metrics	TLBO	SSA	SCA	WOA	BOA	LSHADE	LSHADE-c	DLGWO
*f*_1_	Mean	0.00*E* + 00	4.66*E* − 09	3.46*E* − 43	0.00*E* + 00	1.42*E* − 10	0.00*E* + 00	0.00*E* + 00	0.00*E* + 00
	SD	0.00*E* + 00	1.19*E* − 09	6.93*E* − 43	0.00*E* + 00	5.65*E* − 12	0.00*E* + 00	0.00*E* + 00	0.00*E* + 00
	Rank	1	6	5	1	7	1	1	1
*f*_2_	Mean	0.00*E* + 00	3.81*E* − 03	4.93*E* − 46	0.00*E* + 00	4.77*E* − 08	0.00*E* + 00	0.00*E* + 00	0.00*E* + 00
	SD	0.00*E* + 00	6.26*E* − 03	9.66*E* − 46	0.00*E* + 00	3.81*E* − 09	0.00*E* + 00	0.00*E* + 00	0.00*E* + 00
	Rank	1	7	6	1	8	1	1	1
*f*_3_	Mean	3.52*E* − 145	6.23*E* − 08	1.73*E* − 01	1.81*E* + 00	1.15*E* − 10	0.00*E* + 00	0.00*E* + 00	6.22*E* − 181
	SD	4.05*E* − 145	1.75*E* − 08	2.04*E* − 01	3.30*E* − 01	5.43*E* − 12	0.00*E* + 00	0.00*E* + 00	4.26*E* − 182
	Rank	4	6	7	8	5	1	1	3
*f*_4_	Mean	4.19*E* − 122	1.92*E* − 02	2.07*E* − 04	1.94*E* − 02	6.43*E* − 08	2.39*E* − 55	2.46*E* − 72	9.57*E* − 148
	SD	2.06*E* − 122	4.36*E* − 03	3.67*E* − 04	3.88*E* − 03	2.25*E* − 09	7.58*E* − 56	1.22*E* − 72	1.04*E* − 149
	Rank	2	7	6	8	5	4	3	1
*f*_5_	Mean	2.39*E* + 01	9.34*E* + 01	2.75*E* + 01	2.46*E* + 01	2.38*E* + 01	1.74*E* + 00	5.52*E* + 00	2.36*E* + 01
	SD	1.84*E* − 01	7.11*E* + 01	7.45*E* − 01	3.79*E* − 01	1.57*E* + 00	9.29*E* − 01	1.05*E* + 00	3.88*E* − 01
	Rank	5	8	7	6	4	1	2	3
*f*_6_	Mean	4.19*E* − 22	3.55*E* − 09	4.70*E* − 01	3.74*E* − 06	3.74*E* − 01	0.00*E* + 00	0.00*E* + 00	5.05*E* − 07
	SD	5.65*E* − 22	1.02*E* − 09	2.62*E* − 02	1.67*E* − 06	2.82*E* − 01	0.00*E* + 00	0.00*E* + 00	2.36*E* − 07
	Rank	3	4	8	6	7	1	1	5
*f*_7_	Mean	1.66*E* − 04	2.13*E* − 03	9.19*E* − 03	1.92*E* − 04	2.90*E* − 02	1.75*E* − 03	1.33*E* − 04	2.20*E* − 05
	SD	3.71*E* − 05	1.23*E* − 04	3.52*E* − 03	2.92*E* − 04	2.13*E* − 03	8.52*E* − 04	2.21*E* − 04	7.65*E* − 05
	Rank	3	6	7	5	8	4	2	1
Average rank for *f*_1_ − *f*_7_		2.71	6.28	6.57	5.00	6.28	1.85	1.57	2.14
Final rank for *f*_1_ − *f*_7_		4	6	8	5	6	2	1	3

The article "Dimensional Learning Strategy-Based Grey Wolf Optimizer for Solving the Global Optimization Problem" was published in 2022. Journal: Comput Intell Neurosci.

**Table 12:** Results on benchmark functions *f*_8_–*f*_13_.

	Metrics	TLBO	SSA	SCA	WOA	BOA	LSHADE	LSHADE-c	DLGWO
*f*_8_	Mean	−7.24*E* + 03	−7.80*E* + 03	−6.40*E* + 03	−1.23*E* + 04	−7.06*E* + 03	−7.95*E* + 03	−7.22*E* + 03	−8.29*E* + 03
	SD	6.11*E* + 02	1.01*E* + 03	1.74*E* + 02	3.41*E* + 02	3.29*E* + 02	6.78*E* + 02	5.22*E* + 02	9.02*E* + 02
	Rank	5	4	8	1	7	3	6	2
*f*_9_	Mean	5.55*E* + 00	5.17*E* + 01	0.00*E* + 00	0.00*E* + 00	1.80*E* + 02	0.00*E* + 00	0.00*E* + 00	0.00*E* + 00
	SD	2.26*E* − 01	2.15*E* + 01	0.00*E* + 00	0.00*E* + 00	1.09*E* + 02	0.00*E* + 00	0.00*E* + 00	0.00*E* + 00
	Rank	6	7	1	1	8	1	1	1
*f*_10_	Mean	5.62*E* − 15	1.69*E* + 00	7.99*E* − 15	2.66*E* − 15	1.96*E* + 01	8.88*E* − 16	8.88*E* − 16	4.64*E* − 15
	SD	2.05*E* − 15	7.71*E* − 01	7.20*E* − 15	2.05*E* − 15	6.23*E* − 01	3.49*E* − 16	2.02*E* − 16	1.58*E* − 15
	Rank	5	7	6	3	8	2	1	4
*f*_11_	Mean	0.00*E* + 00	1.14*E* − 02	0.00*E* + 00	0.00*E* + 00	8.57*E* − 11	0.00*E* + 00	0.00*E* + 00	0.00*E* + 00
	SD	0.00*E* + 00	2.83*E* − 03	0.00*E* + 00	0.00*E* + 00	2.84*E* − 11	0.00*E* + 00	0.00*E* + 00	0.00*E* + 00
	Rank	1	8	1	1	7	1	1	1
*f*_12_	Mean	2.45*E* − 24	1.73*E* − 01	3.24*E* − 01	1.12*E* − 06	1.10*E* − 01	2.21*E* − 08	9.26*E* − 09	1.79*E* − 08
	SD	3.77*E* − 24	2.99*E* − 01	1.87*E* − 01	1.03*E* − 07	6.29*E* − 02	7.55*E* − 08	8.24*E* − 10	4.81*E* − 09
	Rank	1	7	8	5	6	4	2	3
*f*_13_	Mean	8.37*E* − 02	1.09*E* − 10	2.06*E* + 00	1.23*E* − 05	1.85*E* + 00	8.89*E* − 07	1.62*E* − 10	2.40*E* − 07
	SD	7.45*E* − 02	3.82*E* − 11	1.05*E* − 01	5.28*E* − 06	4.43*E* − 01	4.55*E* − 08	2.34*E* − 10	7.22*E* − 08
	Rank	6	1	8	5	7	4	2	3
Average rank for *f*_8_ − *f*_13_		4.00	5.67	5.33	2.66	7.17	2.50	2.17	2.33
Final rank for *f*_8_ − *f*_13_		5	7	6	4	8	3	1	2

The article "Dimensional Learning Strategy-Based Grey Wolf Optimizer for Solving the Global Optimization Problem" was published in 2022. Journal: Comput Intell Neurosci.

**Table 13:** Results on benchmark functions *f*_14_–*f*_23_.

	Metrics	TLBO	SSA	SCA	WOA	BOA	LSHADE	LSHADE-c	DLGWO
*f*_14_	Mean	1.02*E* + 00	9.98*E* − 01	9.98*E* − 01	3.43*E* + 00	1.24*E* + 00	1.01*E* + 00	9.98*E* − 01	9.98*E* − 01
	SD	6.21*E* − 01	1.35*E* − 16	4.30*E* − 09	4.88*E* + 00	4.97*E* − 01	4.12*E* − 01	2.24*E* − 15	3.78*E* − 13
	Rank	6	1	4	8	7	5	2	3
*f*_15_	Mean	7.42*E* − 04	1.22*E* − 03	3.19*E* − 04	3.14*E* − 04	3.09*E* − 04	4.85*E* − 05	2.11*E* − 07	3.10*E* − 04
	SD	3.81*E* − 04	2.64*E* − 16	9.75*E* − 06	1.08*E* − 05	1.30*E* − 06	2.21*E* − 05	6.44*E* − 07	3.41*E* − 10
	Rank	7	8	6	5	3	2	1	4
*f*_16_	Mean	−1.03*E* + 00	−1.03*E* + 00	−1.03*E* + 00	−1.03*E* + 00	−1.03*E* + 00	−1.03*E* + 00	−1.03*E* + 00	−1.03*E* + 00
	SD	0.00*E* + 00	2.71*E* − 16	1.09*E* − 06	2.87*E* − 15	3.32*E* − 15	2.11*E* − 09	9.84*E* − 10	1.03*E* − 11
	Rank	1	2	8	3	4	7	6	5
*f*_17_	Mean	3.98*E* − 01	3.98*E* − 01	3.98*E* − 01	3.98*E* − 01	3.98*E* − 01	3.98*E* − 01	3.98*E* − 01	3.98*E* − 01
	SD	0.00*E* + 00	0.00*E* + 00	1.16*E* − 05	2.27*E* − 10	5.06*E* − 05	2.44*E* − 09	7.11*E* − 10	8.29*E* − 10
	Rank	1	1	7	3	8	6	4	5
*f*_18_	Mean	3.00*E* + 00	3.00*E* + 00	3.00*E* + 00	3.00*E* + 00	3.00*E* + 00	3.00*E* + 00	3.00*E* + 00	3.00*E* + 00
	SD	1.33*E* − 15	7.14*E* − 15	2.62*E* − 07	4.09*E* − 09	2.67*E* − 05	0.00*E* + 00	0.00*E* + 00	5.72*E* − 10
	Rank	3	4	7	6	8	1	1	5
*f*_19_	Mean	−3.86*E* + 00	−3.86*E* + 00	−3.85*E* + 00	−3.86*E* + 00	−3.86*E* + 00	−3.86*E* + 00	−3.86*E* + 00	−3.86*E* + 00
	SD	0.00*E* + 00	4.44*E* − 16	6.99*E* − 05	3.94*E* − 03	6.82*E* − 03	5.45*E* − 08	2.72*E* − 06	9.86*E* − 08
	Rank	1	2	6	7	8	3	5	4
*f*_20_	Mean	−3.22*E* + 00	−3.20*E* + 00	−2.98*E* + 00	−3.29*E* + 00	−3.27*E* + 00	−3.30*E* + 00	−3.27*E* + 00	−3.28*E* + 00
	SD	1.55*E* − 02	3.87*E* − 12	3.97*E* − 01	5.98*E* − 02	1.55*E* − 10	1.04*E* − 10	2.55*E* − 08	5.81*E* − 02
	Rank	6	7	8	2	4	1	5	3
*f*_21_	Mean	−9.35*E* + 00	−9.66*E* + 00	−8.92*E* + 00	−1.01*E* + 01	−7.49*E* + 00	−9.94*E* + 00	−1.01*E* + 01	−1.01*E* + 01
	SD	4.32*E* + 00	4.06*E* + 00	2.03*E* + 00	4.55*E* − 07	1.26*E* + 00	3.11*E* − 06	4.15*E* − 05	6.27*E* − 07
	Rank	6	5	7	1	8	4	3	2
*f*_22_	Mean	−9.64*E* + 00	−9.53*E* + 00	−7.03*E* + 00	−1.02*E* + 01	−8.97*E* + 00	−1.02*E* + 00	−9.99*E* + 00	−1.04*E* + *E* + 01
	SD	1.77*E* + 00	1.09*E* + 00	1.71*E* + 00	4.80*E* − 07	2.04*E* + 00	2.85*E* − 07	5.62*E* − 05	7.71*E* − 07
	Rank	5	6	8	3	7	2	4	1
*f*_23_	Mean	−1.02*E* + 00	−9.56*E* + 00	−9.98*E* + 00	−1.02*E* + 01	−7.28*E* + 00	−1.02*E* + 00	−1.02*E* + 00	−1.05*E* + 01
	SD	1.85*E* + 00	2.62*E* + 00	1.56*E* + 00	6.45*E* − 07	1.43*E* + 00	1.92*E* + 00	1.15*E* + 00	2.02*E* − 07
	Rank	4	7	6	2	8	5	3	1
Average rank for *f*_14_ − *f*_23_		4.00	4.30	6.70	4.00	6.50	3.60	3.40	3.30
Final rank for *f*_14_ − *f*_23_		4	6	8	4	7	3	2	1

The article "Dimensional Learning Strategy-Based Grey Wolf Optimizer for Solving the Global Optimization Problem" was published in 2022. Journal: Comput Intell Neurosci.

**Table 14:** Wilcoxon rank-sum test on benchmark functions.

DLGWO vs.	TLBO		SSA		SCA		WOA		BOA		LSHADE		LSHADE-c	
	*p*		*p*		*p*		*p*		*p*		*p*		*p*	
*f*_1_	NaN	≈	NaN	≈	NaN	≈	NaN	≈	NaN	≈	NaN	≈	NaN	≈
*f*_2_	NaN	≈	1.21*E* − 12	+	1.21*E* − 12	+	1.21*E* − 12	+	NaN	≈	NaN	≈	NaN	≈
*f*_3_	4.62*E* − 10	+	1.21*E* − 12	+	1.21*E* − 12	+	1.21*E* − 12	+	1.21*E* − 12	+	2.24*E* − 11	−	2.24*E* − 11	−
*f*_4_	2.20*E* − 09	+	3.02*E* − 11	+	3.02*E* − 11	+	3.02*E* − 11	+	3.02*E* − 11	+	3.02*E* − 11	+	3.02*E* − 11	+
*f*_5_	1.05*E* − 04	+	3.02*E* − 11	+	4.01*E* − 09	+	7.44*E* − 09	+	2.52*E* − 03	+	3.02*E* − 11	−	3.02*E* − 11	−
	7.39*E* − 09	−	5.44*E* − 07	−	3.02*E* − 11	+	1.89*E* − 03	+	3.02*E* − 11	+	3.02*E* − 11	−	3.02*E* − 11	−
*f*_7_	4.52*E* − 02	≈	3.02*E* − 11	+	3.02*E* − 11	+	1.09*E* − 03	+	3.02*E* − 11	+	1.43*E* − 03	+	7.01*E* − 02	≈
*f*_8_	3.02*E* − 11	+	3.02*E* − 11	+	3.02*E* − 11	+	3.02*E* − 11	−	3.02*E* − 11	+	3.02*E* − 11	+	3.02*E* − 11	+
*f*_9_	1.21*E* − 12	+	1.21*E* − 12	+	NaN	≈	NaN	≈	1.21*E* − 12	+	NaN	≈	NaN	≈
*f*_10_	3.02*E* − 11	+	3.02*E* − 11	+	3.02*E* − 11	+	8.22*E* − 07	−	3.02*E* − 11	+	9.22*E* − 09	−	9.22*E* − 09	−
*f*_11_	NaN	≈	1.21*E* − 12	+	NaN	≈	NaN	≈	1.62*E* − 02	≈	NaN	≈	NaN	≈
*f*_12_	3.02*E* − 11	−	3.02*E* − 11	+	3.02*E* − 11	+	2.26*E* − 04	+	3.02*E* − 11	+	4.89*E* − 02	≈	2.72*E* − 02	≈
*f*_13_	5.79*E* − 06	+	8.56*E* − 04	−	2.42*E* − 09	+	3.48*E* − 04	+	3.57*E* − 09	+	1.37*E* − 01	≈	8.79*E* − 04	−
*f*_14_	2.05*E* − 07	+	6.55*E* − 06	−	4.72*E* − 04	+	4.64*E* − 09	+	1.35*E* − 08	+	3.18*E* − 07	+	2.14*E* − 04	−
*f*_15_	1.55*E* − 03	+	3.04*E* − 05	+	6.85*E* − 02	≈	5.36*E* − 02	≈	2.90*E* − 01	≈	2.83*E* − 02	≈	1.28*E* − 03	−
*f*_16_	3.02*E* − 11	−	6.55*E* − 10	−	3.75*E* − 07	+	7.20*E* − 10	−	8.11*E* − 10	−	2.61*E* − 04	+	1.22*E* − 03	+
*f*_17_	1.21*E* − 12	−	1.21*E* − 12	−	5.07*E* − 06	+	4.29*E* − 02	≈	4.10*E* − 06	+	1.22*E* − 02	≈	5.74*E* − 02	≈
*f*_18_	4.24*E* − 07	−	2.27*E* − 06	−	7.02*E* − 04	+	1.74*E* − 02	≈	6.62*E* − 06	+	3.02*E* − 11	−	3.02*E* − 11	−
*f*_19_	3.02*E* − 11	−	4.40*E* − 08	−	6.76*E* − 05	+	1.11*E* − 06	+	6.87*E* − 07	+	4.50*E* − 01	≈	4.08*E* − 03	+
*f*_20_	1.49*E* − 04	+	5.84*E* − 05	+	4.05*E* − 05	+	2.87*E* − 04	−	4.63*E* − 03	+	1.32*E* − 06	−	1.12*E* − 03	+
*f*_21_	6.00*E* − 07	+	4.77*E* − 06	+	3.02*E* − 11	+	2.13*E* − 01	≈	3.02*E* − 11	+	5.91*E* − 03	+	5.24*E* − 01	≈
*f*_22_	6.84*E* − 05	+	1.70*E* − 05	+	1.63*E* − 07	+	1.66*E* − 03	+	6.77*E* − 06	+	2.90*E* − 02	≈	7.40*E* − 04	+
*f*_23_	3.36*E* − 04	+	2.58*E* − 06	+	4.22*E* − 06	+	8.02*E* − 03	+	1.09*E* − 10	+	2.60*E* − 04	+	5.72*E* − 04	+

The article "Dimensional Learning Strategy-Based Grey Wolf Optimizer for Solving the Global Optimization Problem" was published in 2022. Journal: Comput Intell Neurosci.

**Table 15:** Statistical results of the Wilcoxon rank-sum test.

DLGWO vs.		*f*_1_–*f*_7_	*f*_8_–*f*_13_	*f*_14_–*f*_23_	Sum
Wilcoxon's rank-sum test (+/≈/−)	TLBO	3/3/1	4/1/1	6/0/4	13/4/6
	SSA	5/1/1	5/0/1	5/0/5	15/1/7
	SCA	6/1/0	4/2/0	9/1/0	19/4/0
	WOA	6/1/0	2/2/2	4/4/2	12/7/4
	BOA	5/2/0	5/1/0	8/1/1	18/4/1
	LSHADE	2/2/3	1/4/1	4/4/2	7/10/6
	LSHADE-cnEpSin	1/3/3	1/3/2	5/2/3	7/8/8

**Table 16:** Comparison results on the spring design problem.

Algorithms	*x*_1_	*x*_2_	*x*_3_	Optimal cost
DLGWO	0.051260	0.346480	11.916330	0.012670
GWO [25]	0.050149	0.320762	13.757132	0.012711
learnGWO [50]	0.050365	0.325661	13.376170	0.012702
GSA [62]	0.050005	0.317518	14.023225	0.012722
SCA [21]	0.055355	0.451498	7.323204	0.012898
MVO [63]	0.050001	0.317402	14.032308	0.012721
WOA [22]	0.054637	0.431879	7.941518	0.012817
HHO [24]	0.052201	0.369155	10.595956	0.012671
LSHADE [57]	0.051700	0.356979	11.274151	0.012667

**Table 17:** Comparison results on the welded beam problem.

Algorithms	*y*_1_	*y*_2_	*y*_3_	*y*_4_	Optimal cost
DLGWO	0.205729	3.470489	9.036624	0.205729	1.724853
GWO [25]	0.205709	3.469307	9.040968	0.205712	1.725276
RWGWO [39]	0.205519	3.475426	9.036760	0.205753	1.725179
MFO [64]	0.205727	3.470552	9.036614	0.205731	1.724861
KH [65]	0.203720	3.530723	9.036809	0.205838	1.730702
BOA [23]	0.205674	3.474845	9.036501	0.205744	1.725452
SSA [20]	0.204800	3.491382	9.039175	0.205724	1.726626
MPA [66]	0.205666	3.473276	9.041017	0.205726	1.725866
JADE [67]	0.205728	3.470518	9.036617	0.205730	1.724858

**Table 18:** Comparison results on the pressure vessel design problem.

Algorithms	*z*_1_	*z*_2_	*z*_3_	*z*_4_	Optimal cost
DLGWO	0.7785	0.3848	40.3380	199.7643	5886.5293
GWO [25]	0.7791	0.3852	40.3651	199.3867	5887.6935
EEGWO [29]	0.7921	0.3964	40.7491	194.8122	5978.3454
CMA-ES [69]	0.7805	0.3869	40.4375	198.3741	5892.6520
TSO [70]	0.7952	0.4122	41.0635	190.6280	6006.5711
CSA [71]	0.8235	0.4372	42.6094	170.7793	6081.1492
EO [72]	0.7827	0.3878	40.5559	196.7654	5896.5698
TLBO [19]	0.7963	0.4226	41.2309	188.0681	6016.6774
DA [73]	0.7784	0.3855	40.3279	199.9235	5888.7013

## Data Availability

The data used to support the findings of this study are available from the corresponding author upon request.
